# Optimal Combinations of Control Strategies and Cost-Effectiveness Analysis of Dynamics of Endemic Malaria Transmission Model

**DOI:** 10.1155/2023/7677951

**Published:** 2023-05-29

**Authors:** Dereje Gutema Edossa, Alemu Geleta Wedajo, Purnachandra Rao Koya

**Affiliations:** Department of Mathematics, Wollega University, Nekemte, Ethiopia

## Abstract

In this study, we propose and analyze a determinastic nonlinear system of ordinary differential equation model for endemic malaria disease transmission and optimal combinations of control strategies with cost effective analysis. Basic properties of the model, existence of disease-free and endemic equilibrium points, and basic reproduction number of the model are derived and analyzed. From this analysis, we conclude that if the basic reproduction number is less than unity, then the disease-free equilibrium point is both locally and globally asymptotically stable. The endemic equilibrium will also exist if the basic reproduction number is greater than unity. Moreover, existence and necessary condition for forward bifurcation is derived and established. Furthermore, optimal combinations of time-dependent control measures are incorporated to the model. By using Pontryagin's maximum principal theory, we derived the necessary conditions of optimal control. Numerical simulations were conducted to confirm our analytical results. Our findings were that malaria disease may be controlled well with strict application of the combination of prevention of drug resistance, insecticide-treated net (ITN), indoor residual spray (IRS), and active treatment. The use of a combination of insecticide-treated net, indoor residual spray, and active treatment is the most optimal cost-effective and efficacious strategy.

## 1. Introduction

Malaria is an old deadly parasitic disease and transmitted to the human through the bites of infected female *Anopheles* mosquito. It is still treated as a serious challenge to the global world population. According to 2020 World Health Organization (WHO) report, there were 241 million cases and 627 thousand deaths from malaria globally. Specifically, according to the report, 80% of the total deaths occurred in Africa among children aged under 5 years old due to malaria [1].

The most popularly used malaria intervention strategies in sub-Saharan Africa and Asia include the use of insecticide-treated bed net (ITN) and indoor residual spray (IRS) against the vector and treatment of infected individuals with drugs. However, despite intensive control efforts, global incidence of malaria is increasing in malaria endemic area. This is due to one of the factors contributed by the spread and emergence of drug-resistant parasite strains against the most common and affordable antimalarial drugs and resistance of malaria vectors against insecticides in sub-Saharan Africa [2, 3].

Mathematical modeling has become an important tool in understanding the complex dynamics of disease transmission and in decision-making processes regarding intervention programs for disease control. Concerning malaria disease, Ross developed the first mathematical model. He focused his study on mosquito control and showed that for the disease to be eliminated, the mosquito population should be brought below a certain threshold [4]. Later, the idea of Ross is extended by McDonald to account for super infection [5]. Ngwa and Shu are formulated and analyzed a mathematical model for endemic malaria with variable human and mosquito populations [6]. Wedajo et al. derived and analyzed a deterministic model for the inclusion of infected immigrants on the spread and dynamics of malaria transmission [7]. Chiyaka et al. derived and analyzed the effects of treatment and drug resistance on the transmission dynamics of malaria in endemic areas [8]. Tumwiine et al. analyzed a mathematical model for the transmission and spread of drug-sensitive and drug-resistant malaria strains within human populations [9]. Other studies are carried out by using optimal control theory. Okosun et al. derived and analyzed a malaria disease transmission mathematical model that includes treatment and vaccination with waning immunity and applied optimal control to study the impact of a possible vaccination with treatment strategies in controlling the spread of malaria [10]. Agusto and Khan derived and analyzed optimal control strategies for dengue transmission [11]. Okosun and Makinde modeled the impact of drug resistance in malaria transmission and its optimal control analysis [12]. Bonyah et al. present “Modeling the effects of heavy alcohol consumption on the transmission dynamics of gonorrhea with optimal” [13]. Makinde and Okosun applied optimal control to study the impact of chemotherapy on malaria disease with infective immigrants [14]. Okosun et al. applied optimal control strategies and cost-effectiveness analysis of a malaria model [15]. Keno et al. derived and analyzed optimal control and cost effectiveness analysis of SIRS malaria disease model with temperature variability [16].

In this paper, we study SITRS-SI and SIRS-SI endemic malaria transmission model with standard incidence law that was presented by [12]. Furthermore, we modified the model [6] by omitting the incubating class from the system and incorporating four time-dependent control measures, the class infective in treatment individuals and infectious classes with drug-sensitive and drug-resistant individuals. The purpose of this study is to

- investigate the stability for both disease-free equilibrium and endemic equilibrium
- develop effective ways for controlling the malaria disease
- explore the best strategy in terms of reducing the number of malaria infectious populations to zero and minimizing costs

## 2. Model Description and Formulation

To study the transmission and spread of malaria in two interacting population of humans (the host) and mosquitoes (the vector), we formulate a model which subdivides the total human population size at time *t*, denoted by  *N*_*h*_(*t*) into susceptible  *S*_*h*_, infected with drug-sensitive malaria strain  *I*_*hs*_, infected with drug-resistant malaria strain  *I*_*hr*_, infective in treatment *T*_*h*_, and recovered *R*_*h*_. Hence, we have

(1) $$\begin{array}{c} N_{h}\left(t\right)=S_{h}\left(t\right)+I_{hs}\left(t\right)+I_{hr}\left(t\right)+T_{h}\left(t\right)+R_{h}\left(t\right). \end{array}$$

Unlike human population, we divide the mosquito population into two compartments: susceptible  *S*_*v*_ and infected  *I*_*v*_.Thus, the total size of the mosquito population at any time *t* is denoted by

(2) $$\begin{array}{c} \;N_{v}\left(t\right)=S_{v}\left(t\right)+I_{v}\left(t\right). \end{array}$$

Note that  *S*_*h*_ = *S*_*h*_(*t*),  *I*_*hs*_ = *I*_*hs*_(*t*), *I*_*hr*_ = *I*_*hr*_(*t*),  *T*_*h*_ = *T*_*h*_(*t*),  *R*_*h*_ = *R*_*h*_(*t*),  *S*_*v*_ = *S*_*v*_(*t*),  *I*_*v*_ = *I*_*v*_(*t*),  *N*_*v*_ = *N*_*v*_(*t*), and  *N*_*h*_ = *N*_*h*_(*t*), where *ε* denotes the rate of infective in treatment individuals that enter in to the susceptible human compartment due to the administered drug kills off the parasites in his/her body and *θ* represents the rate of recovered individuals that enter in to the susceptible human compartment due to loss of immunity. The susceptible human compartment class is increased due to (i) birth or immigration with a constant requirement rate *Λ*_*h*_; (ii) the administered drug kills off the parasites in the cell of malaria-infected individuals, and these are found in the infective in treatment human compartment class with respective rate *ε*; and (iii) immunity loss of individuals in the recovered human compartment class. This group is further reduced by natural death rate *μ*_*h*_ and per capita rate of force of infection *λ*_*h*_. Hence, the rate of change of the susceptible human compartment class is given by

(3) $$\begin{array}{c} \frac{dS_{h}}{dt}=\Lambda_{h}+\varepsilon T_{h}+\theta R_{h}-\left(\lambda_{h}+\mu_{h}\right)S_{h}. \end{array}$$

Furthermore, the rate of change of  *I*_*hs*_  class is increased by *ρ*(1 − *π*) *λ*_*h*_*S*_*h*_  and decreased by the quantity (*μ*_*h*_ + *δ*_*h*_ + *α* + *γ*_*s*_)*I*_*hs*_, where *μ*_*h*_, *δ*_*h*_, *γ*_*s*_, and *α*  are natural death rate, disease-induced death rate, recovery rate, and the proportion at which *I*_*hs*_ enjoy *T*_*h*_, respectively. *π* is the modification parameter, and *ρ* is the proportionality per capita rate of susceptible humans entering *I*_*hs*_. Thus, the rate of change is given by

(4) $$\begin{array}{c} \frac{dI_{hs}}{dt}=\rho \left(1-\pi \right)\lambda_{h}S_{h}-\left(\mu_{h}+\delta_{h}+\alpha +\gamma_{s}\right)I_{hs}. \end{array}$$

Furthermore, the rate of change of  *I*_*hr*_ class is increased by (1 − (1 − *π*)*ρ*)*λ*_*h*_*S*_*h*_  and decreased by the quantity (*μ*_*h*_ + *δ*_*h*_ + *γ*_*r*_ + *σ*)*I*_*hr*_, where *μ*_*h*_, *δ*_*h*_, *γ*_*s*_, and *σ* are the natural death rate, disease-induced death rate, recovery rate, and proportion at which *I*_*hr*_ enjoy *T*_*h*_, respectively. (1 − *ρ*) is the proportionality per capita rate of susceptible humans entering *I*_*hr*_. Thus, the rate of change is given by

(5) $$\begin{array}{c} \frac{dI_{hr}}{dt}=\left(1-\left(1-\pi \right)\rho \right)\lambda_{h}S_{h}-\left(\mu_{h}+\delta_{h}+\gamma_{r}+\sigma \right)I_{hr}. \end{array}$$

Also, *T*_*h*_ class is increased by *αI*_*hs*_ and *σI*_*hr*_  but decreased by the quantity (*δ*_*h*_ + *μ*_*h*_ + *ε*)*T*_*h*_, where *π*_1_ is the modification parameter and *ε*  is treatment rate. Thus, the rate change of state equation is given by

(6) $$\begin{array}{c} \frac{dT_{h}}{dt}=\alpha I_{hs}+\sigma I_{hr}-\left(\delta_{h}+\mu_{h}+\varepsilon \right)T_{h}. \end{array}$$

The rate of change of the population of the partially immune group (recovered class) *R*_*h*_  is increased by *γ*_*s*_*I*_*hs*_ and *γ*_*r*_*I*_*hr*_ and decreased by the quantity (*θ* + *μ*_*h*_)*R*_*h*_, where *θ* is per capita rate of immunity loss. Thus, the rate change of state equation is given by

(7) $$\begin{array}{c} \frac{dR_{h}}{dt}=\gamma_{s}I_{hs}+\gamma_{r}I_{hr}-\left(\theta +\mu_{h}\right)R_{h}. \end{array}$$

The rate of change of the population of the susceptible mosquito is generated by the recruitment of mosquitos  *Λ*_*v*_ and decreased by the natural death rate *μ*_*v*_*S*_*v*_ and force of infection  *λ*_*v*_*S*_*v*_  between the susceptible and infected classes such that

(8) $$\begin{array}{c} \frac{dS_{v}}{dt}=\Lambda_{v}-\left(\lambda_{v}+\mu_{v}\right)S_{v}. \end{array}$$

Finally, the rate of change of the population of the infected mosquito is generated by the force of infection *λ*_*v*_*S*_*v*_ and decreased by the quantity (*μ*_*v*_ + *δ*_*v*_)*I*_*v*_, where *μ*_*v*_  and *δ*_*v*_  are the natural and disease-induced death rates of the mosquito, respectively. Thus, it is given by

(9) $$\begin{array}{c} \frac{dI_{v}}{dt}=\lambda_{v}S_{v}-\left(\mu_{v}+\delta_{v}\right)I_{v}. \end{array}$$

The notation

(10) $$\begin{array}{c} \;\lambda_{h}=\phi {\omega \beta }_{h}\frac{I_{v}}{N_{h}}, \end{array}$$

where *β*_*h*_ is the rate of probability of human getting infected, *ϕ*  is the mosquito contact rate with human, and  *ω*  is mosquito biting rate.

(11) $$\begin{array}{c} \;\lambda_{v}=\phi \omega \beta_{v}\;\left(\frac{I_{hs}+I_{hr}}{N_{h}}\right), \end{array}$$

where  *β*_*v*_ is the probability of a mosquito getting infected and *σ*_*h*_ is the modification parameter.

Assumptions in the model build-up are as follows:

- The susceptible class in both the human and mosquito populations enters into the infective classes by adequate contact with infectious populations not infective in treatment
- Infective in treatment and recovered individuals are not infectious to the susceptible populations
- Those infective humans recovered from the disease due to natural immunity and enter into a partially immune group
- Those infective individuals in treatment recovered from the disease because the administered drug killed off the parasites
- One part of the recovered class again becomes susceptible to the disease
- No recovered compartment for mosquitoes

We represent the above model description diagrammatically in Figure 1.

Figure 1 can be expressed or written in seven systems of ordinary differential equations as follows:

(12) $$\begin{array}{c} \left\{\begin{array}{c} \frac{dS_{h}}{dt}=\Lambda_{h}+\varepsilon T_{h}+\theta R_{h}-\left(\lambda_{h}+\mu_{h}\right)S_{h},\\ \frac{dI_{hs}}{dt}=\rho \left(1-\pi \right)\lambda_{h}S_{h}-\left(\mu_{h}+\delta_{h}+\alpha +\gamma_{s}\right)I_{hs},\\ \frac{dI_{hr}}{dt}=\left(1-\left(1-\pi \right)\rho \right)\lambda_{h}S_{h}-\left(\mu_{h}+\delta_{h}+\gamma_{r}+\sigma_{r}\right)I_{hr,}\\ \frac{dT_{h}}{dt}=\alpha I_{hs}+\sigma_{r}I_{hr}-\left(\delta_{h}+\mu_{h}+\varepsilon \right)T_{h},\\ \frac{dR_{h}}{dt}=\gamma_{s}I_{hs}+\gamma_{r}I_{hr}-\left(\theta +\mu_{h}\right)R_{h,}\\ \frac{dS_{v}}{dt}=\Lambda_{v}-\left(\lambda_{v}+\mu_{v}\right)S_{v},\\ \frac{dI_{v}}{dt}=\lambda_{v}{\text{S}}_{v}-\left(\mu_{v}+\delta_{v}\right)I_{v}, \end{array}\;\right. \end{array}$$

with initial conditions

(13) $$\begin{array}{c} S_{h}\left(0\right)=S_{0h},\\ I_{hs}\left(0\right)=I_{0hs},\\ I_{hr}\left(0\right)=I_{0hr},\\ T_{h}\left(0\right)=T_{0h},\\ R_{h}\left(0\right)=R_{0h},\\ S_{v}\left(0\right)=S_{0v},\\ I_{v}\left(0\right)=I_{0v}. \end{array}$$

## 3. Model Analysis

### 3.1. Invariant Region

**Theorem 1 .**

The feasible region *Ω* is defined by *Ω* = {*Ω*_h_ × *Ω*_v_} ⊂ {(*S*_*h*_ *I*_hs_,  *I*_hr_,  *T*_*h*_,  *R*_*h*_,  *S*_*v*_,  *I*_*v*_) ∈ ℝ_+_^7^ : N_h_ ≤ *Λ*_*h*_/*μ*_*h*_ and N_v_ ≤ *Λ*_*v*_/*μ*_*v*_ }; here, $\Omega_{\text{h}}=\left\{\left(\begin{array}{ccccc} S_{h} & I_{\text{hs}}, & I_{\text{hr}}, & T_{h}, & R_{h} \end{array}\right)\in {\mathbb{R}}_{+}^{5}:{\text{N}}_{\text{h}}\leq \Lambda_{h}/\mu_{h}\right\}$ and $\Omega_{\text{v}}=\left\{\left(\begin{array}{cc} {\text{S}}_{\text{v}}, & {\text{I}}_{\text{v}} \end{array}\right)\;\epsilon \;{\mathbb{R}}_{+}^{2}:{\text{N}}_{\text{v}}\leq \Lambda_{v}/\mu_{v}\right\}$ with initial conditions *S*_0*h*_ > 0, *I*_0hs_(0) > 0, *I*_0hr_(0) > 0, *T*_0*h*_(0) > 0, *R*_0*h*_(0) > 0, and *S*_0*v*_(0) > 0, *I*_0*v*_(0) > 0 that are positively invariant.

**Proof**

The total human population at time *t* is given by  *N*_*h*_ = *S*_*h*_ + *I*_hs_ + *I*_hr_ + *T*_*h*_ + *R*_*h*_.

After differentiating both sides of  *N*_*h*_,

(14) $$\begin{array}{c} \frac{dN_{h}}{dt}=\frac{dS_{h}}{dt}+\frac{dI_{\text{hs}}}{dt}+\frac{dI_{r}}{dt}+\frac{dT_{h}}{dt}+\frac{dR_{h}}{dt}, \end{array}$$

which gives

(15) $$\begin{array}{c} \frac{dN_{h}}{dt}=\Lambda_{h}-\mu_{h}N_{h}-\delta_{h}\left(I_{\text{hs}}+I_{\text{hr}}+T_{h}\right). \end{array}$$

In the absence of mortality due to malaria, equation (15) becomes

(16) $$\begin{array}{c} \frac{\;dN_{h}}{dt}\leq \Lambda_{h}-\mu_{h}N_{h}. \end{array}$$

Equation (16) is equivalent to

(17) $$\begin{array}{c} \frac{dN_{h}}{dt}+\mu_{h}N_{h}\leq \Lambda_{h}. \end{array}$$

The resulting differential inequality can be solved by separation of variables to give

(18) $$\begin{array}{c} \int \frac{d}{dt}\left(N_{h}e^{\mu_{h}t}\right)\leq \int \Lambda_{\text{h}}e^{\mu_{h}t}. \end{array}$$

Taking the initial conditions *t* = 0 and denoting *N*_*h*_(0) by  *N*_0*h*_, then the complete solution is given by

(19) $$\begin{array}{c} \;N_{h}\leq \frac{\Lambda_{h}}{\mu_{h}}+\left(N_{0h}-\frac{\Lambda_{h}}{\mu_{h}}\right)e^{-\mu_{h}t}. \end{array}$$

As *t*⟶∞,

(20) $$\begin{array}{c} 0<N_{h}\leq \frac{\Lambda_{h}}{\mu_{h}}. \end{array}$$

So, if  *N*_0*h*_ ≤ *Λ*_*h*_/*μ*_*h*_, then

(21) $$\begin{array}{c} \underset{t⟶\infty }{\lim}\;N_{h}\leq \frac{\Lambda_{h}}{\mu_{h}}. \end{array}$$

On the other hand, if  *N*_0*h*_ > *Λ*_*h*_/*μ*_*h*_, then

(22) $$\begin{array}{c} N_{h}≅\frac{\Lambda_{h}}{\mu_{h}}. \end{array}$$

From (20)–(22), we have

(23) $$\begin{array}{c} \;N_{0h}\leq N_{h}\left(t\right)\leq \frac{\Lambda_{h}}{\mu_{h}}. \end{array}$$

Thus, the total human population is bounded in the region:

(24) $$\begin{array}{c} \Omega_{\text{h}}=\left\{\left(\begin{array}{ccccc} S_{h} & I_{hs}, & I_{hr}, & T_{h}, & R_{h} \end{array}\right)\in {\mathbb{R}}_{+}^{5}:N_{h}\leq \frac{\Lambda_{h}}{\mu_{h}}\right\}. \end{array}$$

The total mosquito population at time *t* is given by  *N*_*v*_ = *S*_*v*_ + *I*_*v*_.

After differentiating both sides of  *N*_*v*_,

(25) $$\begin{array}{c} \frac{dN_{v}}{dt}=\frac{dS_{v}}{dt}+\frac{dI_{v}}{dt}, \end{array}$$

which gives

(26) $$\begin{array}{c} \frac{dN_{v}}{dt}=\Lambda_{v}-\mu_{v}N_{v}-\delta_{v}I_{v}. \end{array}$$

In the absence of mortality due to malaria, equation (26) becomes

(27) $$\begin{array}{c} \frac{\;dN_{h}}{dt}\leq \Lambda_{v}-\mu_{v}N_{v}. \end{array}$$

Equation (27) is equivalent to

(28) $$\begin{array}{c} \frac{dN_{v}}{dt}+\mu_{v}N_{v}\leq \Lambda_{v}. \end{array}$$

The resulting differential inequality can be solved by separation of variables to give

(29) $$\begin{array}{c} \int \frac{d}{dt}\left(N_{v}e^{\mu_{h}t}\right)\leq \int \Lambda_{v}e^{\mu_{h}t}. \end{array}$$

Taking the initial conditions *t* = 0 and denoting *N*_*v*_(0) by  *N*_0*v*_, then the complete solution is given by

(30) $$\begin{array}{c} \;N_{v}\leq \frac{\Lambda_{v}}{\mu_{v}}+\left(N_{0v}-\frac{\Lambda_{v}}{\mu_{v}}\right)e^{-\mu_{v}t}. \end{array}$$

As *t*⟶∞,

(31) $$\begin{array}{c} 0<N_{v}\leq \frac{\Lambda_{v}}{\mu_{v}}. \end{array}$$

So, if  *N*_0*v*_ ≤ *Λ*_*v*_/*μ*_*v*_ , then

(32) $$\begin{array}{c} \underset{t⟶\infty }{\lim}N_{v}\leq \frac{\Lambda_{v}}{\mu_{v}}. \end{array}$$

On the other hand, if  *N*_0*v*_ > *Λ*_*v*_/*μ*_*v*_, then

(33) $$\begin{array}{c} N_{v}≅\frac{\Lambda_{v}}{\mu_{v}}. \end{array}$$

From equations (31)–(33), we have

(34) $$\begin{array}{c} N_{0v}\leq N_{v}\leq \frac{\Lambda_{v}}{\mu_{v}}. \end{array}$$

Thus, the total mosquito population is bounded in the region:

(35) $$\begin{array}{c} \Omega_{v}=\left\{\left(\begin{array}{cc} S_{v}, & I_{v} \end{array},\right)\epsilon {\mathbb{R}}_{+}^{2}:N_{v}\leq \frac{\Lambda_{v}}{\mu_{v}}\right\}. \end{array}$$

Thus, the feasible solution set of the system equation of the model enters and remains in the region:

(36) $$\begin{array}{c} \Omega =\left\{\left(\begin{array}{ccccccc} S_{h}, & I_{hs}, & I_{hr}, & T_{h}, & R_{h}, & S_{v}, & I_{v} \end{array}\right)\in {\mathbb{R}}_{+}^{7}:N_{h}\leq \frac{\Lambda_{h}}{\mu_{h}}\text{ and }N_{v}\leq \frac{\Lambda_{v}}{\mu_{v}}\right\}. \end{array}$$

Therefore, the basic model (12) is well posed epidemiologically and mathematically. Hence, it is sufficient to study the dynamics of the basic model in *Ω*.

### 3.2. Positivity of Solutions

In this section, we aim to obtain nonnegative solutions when dealing with human populations. Therefore, the next discussion below targets on the conditions under which the model being studied has nonnegative solutions.

**Theorem 2 .**

Every solution of the model (12) with initial condition (13) exists in the interval [0, ∞) and *S*_*h*_(*t*) > 0, *I*_*hs*_(*t*) > 0, *I*_*hr*_(*t*) > 0, *T*_*h*_(*t*) > 0, *R*_*h*_(*t*) > 0, *S*_*v*_(*t*) > 0, and  *I*_*v*_(*t*) > 0  for all *t* ≥ 0.

**Proof**

To show the positivity of solutions, it is enough to show that each of the trajectories of system (12) is nonnegative for all *t* ≥ 0.

Since the right-hand side of system (12) is completely continuous and locally Lipschitzian on *C*^1^, the solution  (*S*_*h*_(*t*), *I*_*hs*_(*t*), *I*_*hr*_(*t*), *T*_*h*_(*t*), *R*_*h*_(*t*), *S*_*v*_(*t*), *I*_*v*_(*t*)) of system (12) with initial condition equation (13) exists and is unique on [0, *k*), where 0 < *k* < +∞.

It follows from equation (3) that the differential inequality describing the evolution of the susceptible human population over time *t* is given by

(37) $$\begin{array}{c} \frac{dS_{h}}{dt}\geq \Lambda_{h}-\left(\phi {\omega \beta }_{h}\left(\frac{I_{v}}{N_{h}}\right)\left(t\right)+\mu_{h}\right)S_{h}\left(t\right),\\ \frac{d}{dt}\left[S_{h}\left(t\right)\exp\left\{\mu_{h}t+\int_{0}^{t}\phi {\omega \beta }_{h}\left(\frac{I_{v}}{N_{h}}\right)\left(s\right)ds\right\}\right]\geq \Lambda_{h}\exp\left\{\mu_{h}t+\int_{0}^{t}\phi {\omega \beta }_{h}\left(\frac{I_{v}}{N_{h}}\right)\left(s\right)ds\right\}. \end{array}$$

Hence,

(38) $$\begin{array}{c} S_{h}\left(t\right)\exp\left\{\mu_{h}t+\int_{0}^{t}\phi {\omega \beta }_{h}\left(\frac{I_{v}}{N_{h}}\right)\left(s\right)ds\right\}-S_{0h}\geq \int_{\tilde{t}}^{t}\Lambda_{h}\exp\left\{\mu_{h}t+\int_{0}^{t}\phi {\omega \beta }_{h}\left(\frac{I_{v}}{N_{h}}\right)\left(\psi \right)d\psi \right\}dt. \end{array}$$

Thus,

(39) $$\begin{array}{c} S_{h}\left(t\right)\geq S_{0h}\exp\left[-\left\{\mu_{h}t+\int_{0}^{t}\phi {\omega \beta }_{h}\left(\frac{I_{v}}{N_{h}}\right)\left(S_{h}\right)ds\right\}\right]+\exp\left[-\left\{\mu_{h}t+\int_{0}^{t}\phi {\omega \beta }_{h}\left(\frac{I_{v}}{N_{h}}\right)\left(s\right)ds\right\}\right]\times \int_{0}^{t}\Lambda_{h}\exp\left\{\mu_{h}t+\int_{0}^{t}\phi {\omega \beta }_{h}\left(\frac{I_{v}}{N_{h}}\right)\left(\psi \right)d\psi \right\}dt>0. \end{array}$$

From equation (4), we have (*dI*_*h*_)/*dt* ≥ −(*μ*_*h*_ + *δ*_*h*_ + *α* + *γ*_*s*_)*I*_*hs*_(*t*) that is equivalent to *I*_*hs*_(*t*) ≥ exp[−(*μ*_*h*_ + *δ*_*h*_ + *α* + *γ*_*s*_)*t*] > 0.

From equation (5), we have (*dI*_*h*_)/*dt* ≥ −(*μ*_*h*_ + *δ*_*h*_ + *σ*_*r*_ + *γ*_*r*_)*I*_*hr*_(*t*) that is equivalent to *I*_*hs*_(*t*) ≥ exp[−(*μ*_*h*_ + *δ*_*h*_ + *σ*_*r*_ + *γ*_*r*_)*t*] > 0.

From equation (6), we have (*dT*_*h*_)/*dt* ≥ −(*μ*_*h*_ + *δ*_*h*_ + *ϵ*)*I*_*h*_(*t*) that is equivalent to *T*_*h*_(*t*) ≥ exp[−(*μ*_*h*_ + *δ*_*h*_ + *ε*)*t*] > 0.

From equation (7), we have (*dR*_*h*_)/*dt* ≥ −(*μ*_*h*_ + *θ*)*I*_*h*_(*t*) that is equivalent to *R*_*h*_(*t*) ≥ exp[−(*μ*_*h*_ + *θ*)*t*] > 0.

From equation (8), we have

(40) $$\begin{array}{c} \frac{dS_{v}}{dt}\geq \Lambda_{v}-\left(\int_{0}^{t}\phi {\omega \beta }_{v}\left(\frac{I_{\text{hs}}+I_{\text{hr}}}{N_{h}}\right)\left(t\right)+\mu_{v}\right)S_{v},\\ \frac{d}{dt}\left[S_{v}\left(t\right)\exp\left\{\mu_{\text{v}}t+\int_{0}^{t}\phi {\omega \beta }_{v}\left(\frac{I_{\text{hs}}+I_{\text{hr}}}{N_{h}}\right)\left(s\right)ds\right\}\right]\geq \Lambda_{v}\exp\left\{\mu_{h}t+\int_{0}^{t}\phi {\omega \beta }_{v}\left(\frac{I_{\text{hs}}+I_{\text{hr}}}{N_{h}}\right)\left(s\right)ds\right\}. \end{array}$$

Hence,

(41) $$\begin{array}{c} S_{v}\left(t\right)\exp\left\{\mu_{v}t+\int_{0}^{t}\phi {\omega \beta }_{v}\left(\frac{I_{\text{hs}}+I_{\text{hr}}}{N_{h}}\right)\left(s\right)ds\right\}-S_{0v}\geq \int_{\tilde{t}}^{t}\Lambda_{v}\exp\left\{\mu_{v}t+\int_{0}^{t}\phi {\omega \beta }_{v}\left(\frac{I_{\text{hs}}+I_{\text{hr}}}{N_{h}}\right)\left(\psi \right)d\psi \right\}dt. \end{array}$$

Thus,

(42) $$\begin{array}{c} S_{v}\left(t\right)\geq S_{0h}\exp\left[-\left\{\mu_{v}t+\int_{0}^{t}\phi {\omega \beta }_{v}\left(\frac{I_{\text{hs}}+I_{\text{hr}}}{N_{h}}\right)\left(s\right)ds\right\}\right]+\exp\left[-\left\{\mu_{v}t+\int_{0}^{t}\phi {\omega \beta }_{h}\left(\frac{I_{\text{hs}}+I_{\text{hr}}}{N_{h}}\right)\left(s\right)ds\right\}\right]\times \int_{0}^{t}\Lambda_{v}\exp\left\{\mu_{v}t+\int_{0}^{t}\phi {\omega \beta }_{v}\left(\frac{I_{hs}+I_{hr}}{N_{h}}\right)\left(\psi \right)d\psi \right\}dt>0. \end{array}$$

From equation (9), we have (*dI*_*v*_)/*dt* ≥ −(*μ*_*v*_ + *δ*_*v*_)*I*_*v*_(*t*) that is equivalent to *I*_*v*_(*t*) ≥ exp[−(*μ*_*v*_ + *δ*_*v*_)*t*] > 0.

Therefore, we can see that *S*_*h*_(*t*) > 0, *I*_*hs*_(*t*) > 0, *I*_*hr*_(*t*) > 0, *T*_*h*_(*t*) > 0, *R*_*h*_(*t*) > 0, *S*_*v*_(*t*) > 0, and  *I*_*v*_(*t*) > 0 for all *t* ≥ 0.

### 3.3. Disease-Free Equilibrium (DFE)

In this section, we establish the existence of the disease-free equilibrium point of system (12). The disease-free equilibrium point of the model is its steady-state solutions without infection or disease. Let the right-hand side of equation (12) equal to zero, that is,

(43) $$\begin{array}{c} \frac{dS_{h}}{dt}=\frac{dI_{\text{hs}}}{dt}=\frac{dI_{\text{hr}}}{dt}=\frac{dT_{h}}{dt}=\frac{dR_{h}}{dt}=\frac{dS_{v}}{dt}=\frac{dI_{v}}{dt}=0. \end{array}$$

Then, system (12) becomes

(44) $$\begin{array}{c} \left.\begin{array}{c} \Lambda_{h}+\varepsilon T_{h}+\theta R_{h}-\left(\lambda_{h}+\mu_{h}\right)S_{h}=0,\\ \rho \left(1-\pi \right)\lambda_{h}S_{h}-\left(\mu_{h}+\delta_{h}+\alpha +\gamma_{s}\right)I_{hs}=0,\\ \left(1-\left(1-\pi \right)\rho \right)\lambda_{h}S_{h}-\left(\mu_{h}+\delta_{h}+\sigma_{r}+\gamma_{r}\right)I_{hr}=0,\\ \alpha I_{hs}+\sigma I_{hr}-\left(\delta_{h}+\mu_{h}+\varepsilon \right)T_{h}=0,\\ \gamma_{s}I_{hs}+\gamma_{r}I_{hr}-\left(\theta +\mu_{h}\right)R_{h}=0,\\ \Lambda_{v}-\left(\lambda_{v}+\mu_{v}\right)S_{v}=0,\\ \lambda_{v}S_{v}-\left(\mu_{v}+\delta_{v}\right)I_{v}=0. \end{array}\right\} \end{array}$$

Again letting  *I*_*hs*_ = *I*_*hr*_ = *T*_*h*_ = *R*_*h*_ = *I*_*v*_ = 0, then (44) leads to

(45) $$\begin{array}{c} \Lambda_{h}-\mu_{h}S_{h}^{0}=0, \end{array}$$

(46) $$\begin{array}{c} \Lambda_{v}-\mu_{v}S_{v}^{0}=0. \end{array}$$

Then by rearranging equations (45) and (46) and after substituting each other, we got

(47) $$\begin{array}{c} S_{h}^{0}=\frac{\Lambda_{h}}{\mu_{h}},\\ S_{v}^{0}=\frac{\Lambda_{v}}{\mu_{v}}. \end{array}$$

Then, the disease-free equilibrium point is given by

(48) $$\begin{array}{c} F_{0}=\left(\begin{array}{cccccc} \frac{\Lambda_{h}}{\mu_{h}} & 0 & 0 & 0 & 0 & \begin{array}{cc} \frac{\Lambda_{v}}{\mu_{v}} & 0 \end{array} \end{array}\right). \end{array}$$

### 3.4. The Basic Reproductive Number (*R*_0_)

In this section, we will determine the threshold parameter that governs the spread of the disease which is called basic reproduction number. To obtain the basic reproduction number *R*_0_ of model (12), we used the next-generation matrix method so that it is the spectral radius of the next-generation matrix [17, 18].

The model equations are rewritten starting with newly infective classes:

(49) $$\begin{array}{c} \left.\begin{array}{c} \frac{dI_{hs}}{dt}=\rho \left(1-\pi \right)\phi {\omega \beta }_{h}\left(\frac{I_{v}}{N_{h}}\right)S_{h}-\left(\mu_{h}+\delta_{h}+\alpha +\gamma_{s}\right)I_{hs},\\ \frac{dI_{hr}}{dt}=\left(1-\left(1-\pi \right)\rho \right)\frac{\phi \omega \beta_{h}I_{v}}{N_{h}}S_{h}-\left(\mu_{h}+\delta_{h}+\sigma_{r}+\gamma_{r}\right)I_{hr},\\ \frac{dI_{v}}{dt}=\phi {\omega \beta }_{v}\left(\frac{I_{hs}+I_{hr}}{N_{h}}\right)S_{v}-\left(\mu_{v}+\delta_{v}\right)I_{v}. \end{array}\right\} \end{array}$$

Let $X_{i}={\left(\begin{array}{ccc} I_{hs} & I_{hr} & \begin{array}{c} I_{v} \end{array} \end{array}\right)}^{T}$, *i* = 1, 2, 3, and *X*_1_ = *I*_*h*s_, *X*_2_ = *I*_*hr*_, and  *X*_3_ = *I*_*v*_; then, by the principle of the next-generation matrix, we can obtain

(50) $$\begin{array}{c} F\left(X_{i}\right)=\left(\begin{array}{c} \rho \left(1-\pi \right)\phi {\omega \beta }_{h}\left(\frac{I_{v}}{N_{h}}\right)S_{h}\\ \left(1-\left(1-\pi \right)\rho \right)\frac{\phi \omega \beta_{h}I_{v}}{N_{h}}S_{h}\\ \phi {\omega \beta }_{v}\left(\frac{I_{hs}+I_{hr}}{N_{h}}\right)S_{v} \end{array}\right),\\ V\left(X_{i}\right)=\left(\begin{array}{c} \left(\mu_{h}+\delta_{h}+\alpha +\gamma_{s}\right)I_{hs}\\ \left(\mu_{h}+\delta_{h}+\sigma_{r}+\gamma_{r}\right)I_{hr}\\ \left(\mu_{v}+\delta_{v}\right)I_{v} \end{array}\right). \end{array}$$

The new infection matrix *F* is given by

(51) $$\begin{array}{c} F=\frac{\partial F\left(X_{i}\right)}{\partial X_{i}}\left(E_{0}\right)=\left(\begin{array}{ccc} 0 & 0 & \left(1-\pi \right)\rho \phi \omega \beta_{h}\\ 0 & 0 & \left(1-\left(1-\pi \right)\rho \right)\phi \omega \beta_{h}\\ \frac{\phi \omega \beta_{v}\Lambda_{v}\mu_{h}}{\Lambda_{h}\mu_{v}} & \frac{\phi \omega \beta_{v}\Lambda_{v}\mu_{h}}{\Lambda_{h}\mu_{v}} & 0 \end{array}\right), \end{array}$$

and the transition matrix  *V* is given by

(52) $$\begin{array}{c} V=\frac{\partial V\left(X_{i}\right)}{\partial X_{i}}\left(E_{0}\right)=\left(\begin{array}{ccc} \left(\mu_{h}+\delta_{h}+\alpha +\gamma_{s}\right) & 0 & 0\\ 0 & \left(\mu_{h}+\delta_{h}+\sigma_{r}+\gamma_{r}\right) & 0\\ 0 & 0 & \left(\mu_{v}+\delta_{v}\right) \end{array}\right). \end{array}$$

Thus,

(53) $$\begin{array}{c} {\text{FV}}^{-1}=\left(\begin{array}{ccc} 0 & 0 & \frac{\left(1-\pi \right)\rho \phi \omega \beta_{h}}{\left(\mu_{v}+\delta_{v}\right)}\\ 0 & 0 & \frac{\left(1-\left(1-\pi \right)\rho \right)\phi \omega \beta_{h}}{\mu_{v}+\delta_{v}}\\ \frac{{\phi \omega \beta }_{v}\mu_{h}\Lambda_{v}}{\left(\mu_{h}+\delta_{h}+\alpha +\gamma_{s}\right)\Lambda_{h}\mu_{v}} & \frac{\phi \omega \beta_{v}\Lambda_{v}\mu_{h}\;}{\left(\mu_{h}+\delta_{h}+\sigma_{r}+\gamma_{r}\right)\Lambda_{h}\mu_{v}} & 0 \end{array}\right). \end{array}$$

The eigenvalue of FV^−1^ can be obtained.

(54) $$\begin{array}{c} \left|\begin{array}{ccc} -\lambda & 0 & \frac{\left(1-\pi \right)\rho \phi \omega \beta_{h}}{\left(\mu_{v}+\delta_{v}\right)}\\ 0 & -\lambda & \frac{\left(1-\left(1-\pi \right)\rho \right)\phi \omega \beta_{h}}{\mu_{v}+\delta_{v}}\\ \frac{{\phi \omega \beta }_{v}\mu_{h}\Lambda_{v}}{\left(\mu_{h}+\delta_{h}+\alpha +\gamma_{s}\right)\Lambda_{h}\mu_{v}} & \frac{\phi \omega \beta_{v}\Lambda_{v}\mu_{h}\;}{\left(\mu_{h}+\delta_{h}+\sigma_{r}+\gamma_{r}\right)\Lambda_{h}\mu_{v}} & -\lambda \end{array}\right|=0,\\ -\lambda \left(\lambda^{2}-\left(\frac{\left(1-\left(1-\pi \right)\rho \right)\phi^{2}\omega^{2}\beta_{v}\beta_{h}\Lambda_{v}{\mu_{h}}_{h}}{\left(\mu_{v}+\delta_{v}\right)\left(\mu_{h}+\delta_{h}+\sigma_{r}+\gamma_{r}\right)\Lambda_{h}\mu_{v}}\right)\right)+\left(\frac{\left(1-\pi \right)\rho \phi^{2}\omega^{2}\beta_{v}\beta_{h}\Lambda_{v}{\mu_{h}}_{h}}{\left(\mu_{v}+\delta_{v}\right)\left(\mu_{h}+\delta_{h}+\alpha +\gamma_{s}\right)\Lambda_{h}\mu_{v}}\right)\lambda =0. \end{array}$$

Then, the eigenvalues are

(55) $$\begin{array}{c} \lambda_{1}=0,\\ \lambda^{2}-\left(\frac{\left(1-\left(1-\pi \right)\rho \right)\phi^{2}\omega^{2}\beta_{v}\beta_{h}\Lambda_{v}{\mu_{h}}_{h}}{\left(\mu_{v}+\delta_{v}\right)\left(\mu_{h}+\delta_{h}+\sigma_{r}+\gamma_{r}\right)\Lambda_{h}\mu_{v}}\right)-\left(\frac{\left(1-\pi \right)\rho \phi^{2}\omega^{2}\beta_{v}\beta_{h}\Lambda_{v}{\mu_{h}}_{h}}{\left(\mu_{v}+\delta_{v}\right)\left(\mu_{h}+\delta_{h}+\alpha +\gamma_{s}\right)\Lambda_{h}\mu_{v}}\right)=0,\\ \lambda_{2,3}=\pm \sqrt{\frac{\phi^{2}\omega^{2}\beta_{h}\beta_{v}\mu_{h}\Lambda_{v}\left(\left(\mu_{h}+\delta_{h}+\sigma +\gamma_{r}\right)\rho \left(1-\pi \right)+\left(\mu_{h}+\delta_{h}+\alpha +\gamma_{s}\right)\left(1-\left(1-\pi \right)\rho \right)\right)}{\Lambda_{h}\mu_{v}\left(\mu_{h}+\delta_{h}+\alpha +\gamma_{s}\right)\left(\mu_{h}+\delta_{h}+\sigma_{r}+\gamma_{r}\right)\left(\mu_{v}+\delta_{v}\right)}}. \end{array}$$

From *λ*_1,_, *λ*_2_, and *λ*_3_, the dominant eigenvalue is *λ*_2_. Therefore, the basic reproductive number is given by

(56) $$\begin{array}{c} R_{0}=\sqrt{\frac{\phi^{2}\omega^{2}\beta_{h}\beta_{v}\mu_{h}\Lambda_{v}\left(\left(\mu_{h}+\delta_{h}+\sigma +\gamma_{r}\right)\rho \left(1-\pi \right)+\left(\mu_{h}+\delta_{h}+\alpha +\gamma_{s}\right)\left(1-\left(1-\pi \right)\rho \right)\right)}{\Lambda_{h}\mu_{v}\left(\mu_{h}+\delta_{h}+\alpha +\gamma_{s}\right)\left(\mu_{h}+\delta_{h}+\sigma_{r}+\gamma_{r}\right)\left(\mu_{v}+\delta_{v}\right)}}. \end{array}$$

### 3.5. Local Stability of Disease-Free Equilibrium

**Theorem 3 .**

The disease-free equilibrium point  *F*_0_  of system (12) is locally asymptotically stable if *R*_0_ < 1 and unstable if *R*_0_ > 1.

**Proof**

The local stability of the system is determined by the signs of the eigenvalues, and it is further proved by linearizing to obtain its Jacobian at disease-free steady-state points so that the Jacobian matrix of system (12) at disease-free equilibrium point  *F*_0_ is defined and given by

(57) $$\begin{array}{c} J\left(F_{0}\right)=\left[\begin{array}{ccccccc} -\mu_{h} & 0 & 0 & \varepsilon & \theta & 0 & -k_{17}\\ 0 & -k_{1} & 0 & 0 & 0 & 0 & k_{27}\\ 0 & 0 & -k_{2} & 0 & 0 & 0 & k_{37}\\ 0 & \alpha & \sigma_{r} & -k_{3} & 0 & 0 & 0\\ 0 & \gamma_{s} & \gamma_{r} & 0 & -k_{4} & 0 & 0\\ 0 & -k_{62} & -k_{63} & 0 & 0 & -\mu_{v} & 0\\ 0 & k_{72} & k_{73} & 0 & 0 & 0 & -k_{5} \end{array}\right], \end{array}$$

where *k*_1_ = (*μ*_*h*_ + *δ*_*h*_ + *α* + *γ*_*s*_), *k*_2_ = (*μ*_*h*_ + *δ*_*h*_ + *σ*_*r*_ + *γ*_*r*_),  *k*_3_ = (*μ*_*h*_ + *δ*_*h*_ + *ε*),  *k*_4_ = (*μ*_*h*_ + *θ*), *k*_5_ = (*μ*_*v*_ + *δ*_*v*_), *k*_17_ = *ϕωβ*_*h*_, *k*_27_ = (1 − *π*)*ρϕωβ*_*h*_, and *k*_37_ = (1 − (1 − *π*)*ρ*)*ϕωβ*_*h*_ *k*_62_ = *k*_63_ = *k*_72_ = *k*_73_ = (*ϕωβ*_*v*_*Λ*_*v*_*μ*_*h*_)/(*Λ*_*h*_*μ*_*v*_).

To obtain the eigenvalue of (57), we compute Det (*FV*^−1^ − *λI*) = 0  as follows:

(58) $$\begin{array}{c} \left|\begin{array}{ccccccc} -\mu_{h-\lambda } & 0 & 0 & \varepsilon & \theta & 0 & -k_{17}\\ 0 & -k_{1}-\lambda & 0 & 0 & 0 & 0 & k_{27}\\ 0 & 0 & -k_{2}-\lambda & 0 & 0 & 0 & k_{37}\\ 0 & \alpha & \sigma_{r} & -k_{3}-\lambda & 0 & 0 & 0\\ 0 & \gamma_{s} & \gamma_{r} & 0 & -k_{4}-\lambda & 0 & 0\\ 0 & -k_{62} & -k_{63} & 0 & 0 & -\mu_{v}-\lambda & 0\\ 0 & k_{72} & k_{73} & 0 & 0 & 0 & -k_{5}-\lambda \end{array}\right|=0. \end{array}$$

As the first and sixth columns contain only the diagonal terms which form the two negative eigenvalues, −*μ*_*h*_ and −*μ*_*v*_, the other four eigenvalues can be obtained from the following:

(59) $$\begin{array}{c} \left|\begin{array}{ccccc} -k_{1}-\lambda & 0 & 0 & 0 & k_{27}\\ 0 & -k_{2}-\lambda & 0 & 0 & k_{37}\\ \alpha & \sigma_{r} & -k_{3}-\lambda & 0 & 0\\ \gamma_{s} & \gamma_{r} & 0 & -k_{4}-\lambda & 0\\ k_{72} & k_{73} & 0 & 0 & -k_{5}-\lambda \end{array}\right|=0. \end{array}$$

In the same way, the third and fourth columns contain only the diagonal terms which form the two negative eigenvalues, −*k*_3_ and −*k*_4_, and the other four eigenvalues can be obtained from the following:

(60) $$\begin{array}{c} \left|\begin{array}{ccc} -k_{1}-\lambda & 0 & k_{27}\\ 0 & -k_{2}-\lambda & k_{37}\\ k_{72} & k_{73} & -k_{5}-\lambda \end{array}\right|=0. \end{array}$$

Thus, the eigenvalues of the submatrix are the roots of the characteristic equation

(61) $$\begin{array}{c} a\lambda^{3}+b\lambda^{2}+c\lambda +d=0. \end{array}$$

Here,

(62) $$\begin{array}{c} \left.\begin{array}{c} a=1,\\ b=k_{1}+k_{2}+k_{5},\\ c=k_{2}k_{5}+k_{1}\left(k_{2}+k_{5}\right)-\frac{\phi^{2}\omega^{2}\beta_{h}\beta_{v}\Lambda_{v}\mu_{h}}{\Lambda_{h}\mu_{v}},\\ d=k_{1}k_{2}k_{5}\left(1-R_{0}^{2}\right). \end{array}\right\} \end{array}$$

By the principle of Routh-Hurwitz criteria [19], equation (61) has negative real eigenvalues if and only if *b* > 0, *d* > 0, and *bc* > *d*. Clearly, we see that *b* > 0  because it is the sum of positive variables, but *d* > 0 if and only if  1 − *R*_0_^2^ > 0 which is equivalent to  *R*_0_ < 1, and hence, all the determinant of eigenvalues of equation (57) will have negative real eigenvalues. Therefore, the disease-free equilibrium point *F*_0_  is locally asymptotically stable.

### 3.6. Global Stability of a Disease-Free Equilibrium (DFE)

**Theorem 4 .**

The disease-free equilibrium point  *F*_0_  of system (12) is globally asymptotically stable if *R*_0_ ≤ 1 and unstable if *R*_0_ > 1.

**Proof**

To prove Theorem 4, we consider the Lyapunov function. So let

(63) $$\begin{array}{c} V=k_{5}\left(k_{2}I_{hs}+k_{1}I_{hr}\right)I_{h}+\phi \omega \beta_{h}\left(\rho \left(1-\pi \right)k_{2}+\left(1-\left(1-\pi \right)\rho \right)k_{1}\right)I_{v}. \end{array}$$

Then by differentiating *L*, both sides lead to

(64) $$\begin{array}{c} \frac{dV}{dt}=k_{5}\left(K_{2}\frac{dI_{hs}}{dt}+k_{1}\frac{dI_{hr}}{dt}\right)+\phi \omega \beta_{h}\rho \left(\left(1-\pi \right)k_{2}+\left(1-\left(1-\pi \right)\rho \right)k_{1}\right)\frac{dI_{v}}{dt}. \end{array}$$

After substituting (*dI*_hs_)/*dt*, (*dI*_hr_)/*dt*, and (*dI*_*v*_)/*dt* from (12) into (64) and simplifying it, then we get

(65) $$\begin{array}{c} \frac{dV}{dt}=\frac{\phi^{2}\omega^{2}\beta_{h}\beta_{v}S_{v}^{0}\left(k_{2}\rho \left(1-\pi \right)+k_{1}\left(1-\left(1-\pi \right)\rho \right)\right)\left(I_{hs}+I_{hr}\right)}{S_{h}^{0}}-k_{1}k_{2}k_{5}. \end{array}$$

Since (*dS*_*h*_)/*dt*≤*Λ*_*h*_/*μ*_*h*_  = *S*_*h*_^0^ = *N*_*h*_^0^,  (*dS*_*v*_)/*dt* ≤ *Λ*_*v*_/*μ*_*v*_ = *S*_*v*_^0^ (65) is equivalent to

(66) $$\begin{array}{c} \frac{dV}{dt}=\frac{\phi^{2}\omega^{2}\beta_{h}\beta_{v}\Lambda_{v}\mu_{h}\left(k_{2}\rho \left(1-\pi \right)+k_{1}\left(1-\left(1-\pi \right)\rho \right)\right)\left(I_{hs}+I_{hr}\right)}{\Lambda_{h}\mu_{h}}-k_{1}k_{2}k_{5}. \end{array}$$

Since *R*_0_^2^ = (*ϕ*^2^*ω*^2^*β*_*h*_*β*_*v*_*Λ*_*v*_*μ*_*h*_*k*_2_*ρ*(1 − *π*) + *k*_1_(1 − (1 − *π*)*ρ*))/(*Λ*_*h*_*μ*_*h*_*k*_1_*k*_2_*k*_5_), (66) is also equivalent to

(67) $$\begin{array}{c} \frac{dV}{dt}=k_{1}k_{2}k_{5}\left(R_{0}^{2}-1\right). \end{array}$$

So,  *dV*/*dt* ≤ 0 if (*R*_0_^2^ − 1) ≤ 0 which leads to  *R*_0_ ≤ 1.  *dV*/*dt* = 0 if and only if *I*_*hs*_ = *I*_*hr*_ = 0 or *R*_0_^2^ = 1. Therefore, by LaSalle's invariant principle [20], every solution to equations of model system (12) with initial condition (13) in  *Ω*  approaches to the disease-free equilibrium point  *F*_0_ at time *t* leading to infinity whenever *R*_0_ ≤ 1.

### 3.7. Existence of Endemic Equilibrium (EE)

The endemic equilibrium is denoted by $E^{*}=\left(\begin{array}{ccccc} S_{h}^{*}, & I_{hs}^{*}, & \begin{array}{cc} I_{hr}^{*}, & T_{h}^{*} \end{array}, & R_{h}^{*}, & \begin{array}{cc} S_{v}^{*}, & I_{v}^{*} \end{array} \end{array}\right)$, and it occurs when the disease persists in the community. To obtain it, we equate all the model equations in (12) to zero. Then, we obtain the following:

(68) $$\begin{array}{c} \left.\begin{array}{c} S_{h}^{*}=\frac{k_{1}k_{2}k_{3}k_{4}\Lambda_{h}}{k_{1}k_{2}k_{3}k_{4}\mu_{h}+\left(\mu_{h}p_{3}+p_{4}\right)\lambda_{h}^{*}},\\ I_{hs}^{*}=\frac{\rho \left(1-\pi \right)\lambda_{h}^{*}S_{h}^{*}}{k_{1}},\\ I_{hr}^{*}=\frac{\left(1-\left(1-\pi \right)\rho \right)\lambda_{h}^{*}S_{h}^{*}}{m_{2}},\\ T_{h}^{*}=\frac{\left(k_{2}\rho \alpha \left(1-\pi \right)+\sigma k_{1}\left(1-\left(1-\pi \right)\rho \right)\right)\lambda_{h}^{*}S_{h}^{*}}{k_{1}k_{2}k_{3}},\\ R_{h}^{*}=\frac{\left.\left(\gamma_{s}\left(1-\pi \right)\rho k_{2}+\gamma_{r}\left(1-\left(1-\pi \right)\rho \right)k_{1}\right)\right)\lambda_{h}^{*}S_{h}^{*}}{k_{1}k_{2}k_{4}},\\ S_{v}^{*}=\frac{\Lambda_{v}}{\mu_{v}+\lambda_{v}^{*}},\\ \;I_{v}^{*}=\frac{\Lambda_{v}\lambda_{v}^{*}}{\left(\mu_{v}+\lambda_{v}^{*}\right)k_{4}}, \end{array}\right\} \end{array}$$

(69) $$\begin{array}{c} \lambda_{h}^{*}=\phi \omega \beta_{h}\frac{I_{v}^{*}}{N_{h}^{*}}, \end{array}$$

(70) $$\begin{array}{c} \lambda_{v}^{*}=\phi \omega \beta_{v}\frac{\left(I_{hs}^{*}+I_{hr}^{*}\right)}{N_{h}^{*}}, \end{array}$$

(71) $$\begin{array}{c} N_{h}^{*}=S_{h}^{*}+I_{\text{hs}}^{*}+I_{\text{hr}}^{*}+T_{h}^{*}+R_{h}^{*}. \end{array}$$

Substituting (68) into (70), we get

(72) $$\begin{array}{c} \lambda_{v}^{*}=\frac{\phi \omega \beta_{v}\left(\left(1-\pi \right)\rho k_{2}+\left(1-\left(1-\pi \right)\rho \right)k_{1}\right)k_{1}k_{2}k_{3}k_{4}\lambda_{h}^{*}}{k_{1}k_{2}\left(k_{1}k_{2}k_{3}k_{4}+p\lambda_{h}^{*}\right)}. \end{array}$$

Substuting (68) and (72), respectively, into (69), we get

(73) $$\begin{array}{c} \lambda_{h}^{*}\left(b_{0}{\left(\lambda_{h}^{*}\right)}^{2}+b_{1}\lambda_{h}^{*}+b_{2}\right)=0, \end{array}$$

(74) $$\begin{array}{c} b_{0}=p_{3}k_{1}k_{2}k_{3}k_{4}k_{5}\Lambda_{h}\left(\mu_{v}p_{3}k_{1}k_{2}+\phi \omega \beta_{v}k_{1}k_{2}k_{3}k_{4}\left(\left(1-\pi \right)\rho k_{2}+\left(1-\left(1-\pi \right)\rho \right)k_{1}\right)\right), \end{array}$$

(75) $$\begin{array}{c} b_{1}=\frac{k_{1}k_{2}k_{5}\mu_{v}\Lambda_{h}}{\mu_{h}}\left(R_{c}^{2}-R_{0}^{2}\right), \end{array}$$

(76) $$\begin{array}{c} b_{2}=k_{1}^{4}k_{2}^{4}k_{3}^{3}k_{4}^{3}k_{5}\mu_{v}\Lambda_{h}\left(1-R_{0}^{2}\right), \end{array}$$

where  *R*_0_ is the basic reproduction number given by (4.2) and

(77) $$\begin{array}{c} R_{c}=\sqrt{\frac{\mu_{h}k_{3}k_{4}\left(\phi \omega \beta_{v}k_{1}k_{2}k_{3}k_{4}\left(\left(1-\pi \right)\rho k_{2}+\left(1-\left(1-\pi \right)\rho \right)k_{1}\right)+2\mu_{v}k_{1}k_{2}p_{3}\right)}{k_{1}^{2}k_{2}^{2}k_{3}^{2}k_{4}^{2}\mu_{v}\left(\mu_{h}p_{3}+p_{4}\right)}}, \end{array}$$

(78) $$\begin{array}{c} p_{3}=k_{4}p_{1}+k_{3}p_{2}+{\text{k}}_{3}{\text{k}}_{4}\left(\left(1-\pi \right)\rho m_{2}+\left(1-\left(1-\pi \right)\rho \right)k_{1}\right), \end{array}$$

Equation (72) admits a trivial solution  *λ*_*h*_^∗^ = 0 which corresponds to the disease-free equilibrium point (DFEP). Now, we assume that  *λ*_*h*_^∗^ ≠ 0, and the existence of endemic equilibria is regulated by the quadratic equation *b*_0_(*λ*_*h*_^∗^)^2^ + *b*_1_*λ*_*h*_^∗^ + *b*_2_ = 0. The coefficient *b*_0_ in (73) is always positive, and *b*_2_ is positive if *R*_0_ < 1 and negative if *R*_0_ > 1. So, the sign of *b*_1_ and *b*_2_  will decide about the positive solution of (72). For the case when *R*_0_ > 1, two solutions can be obtained for (72) that are positive and negative. For the case when considering *b*_2_ = 0 if and only if  *R*_0_ = 1, then a solution of the form  *λ*_*h*_^∗^ = (−*b*_1_)/*b*_0_ exists when  *b*_1_ < 0 (*R*_*c*_ < *R*_0_ ). It follows that the number of endemic equilibria of (12) depends on the coefficients *b*_0_, *b*_1_, and *b*_2_ as follows.

**Theorem 5 .**

System (12) has

- a unique endemic equilibrium if  *b*_2_ < 0  if and only if  *R*_0_ > 1
- a unique endemic equilibrium if  *b*_1_ < 0 and  *b*_2_ = 0 or ( *b*_1_ < 0, *b*_2_ > 0 and *b*_1_^2^ 4*b*_0_*b*_2_ = 0 )
- two endemic equilibria if  *b*_2_ > 0 and  *b*_1_ < 0 and *b*_1_^2^ − 4*b*_0_*b*_2_ > 0
- otherwise, no endemic equilibrium

It follows here also that when we put the value of *Λ*_*h*_ = 0.071 and *μ*_*h*_ = 0.115 and use Table 1 for the values of other parameters, the two roots are presented graphically as shown in Figure 2.

From Figure 2, we note that there is stable disease-free region when  *λ*_*h*_^∗^ = 0, and when  *R*_0_ = 1, the force of infection mosquitoes to humans starts to increase in stable endemic region where also the disease starts to spread again and hence forward bifurcation. Here, the blue line represents stable equilibrium, and the red line represents unstable equilibrium.

### 3.8. Existence of Bifurcation

To show the existence of bifurcation of (12), we used the method developed by [21–24]. In these approaches, the center manifold theory was employed to determine the existence and types of bifurcation using the coefficients, *a* and *b*, of the normal form representing the dynamics of the system. These coefficients decide the bifurcation. In particular, if *a* < 0 and *b* > 0, then the bifurcation is forward; if *a* > 0 and *b* > 0, then the bifurcation is backward.

Using this approach, the following result may be obtained.

**Theorem 6 .**

Model equation (12) exhibits a forward bifurcation at *R*_0_ = 1 if the condition  *B*_0_ < 0  is satisfied. Here, *B*_0_  is given by

(79) $$\begin{array}{c} B_{0}=\frac{\phi \omega \beta_{v}\Lambda_{v}z_{1}k_{1}}{\mu_{v}\Lambda_{h}k_{2}}-\left[\frac{z_{1}\Lambda_{h}k_{1}k_{3}k_{4}k_{5}+\Lambda_{v}\phi \omega \beta_{v}\left[{\left(1-\pi \right)}^{2}\rho^{2}k_{2}^{2}k_{3}k_{4}+z_{1}\left(\varepsilon +\theta +2\mu_{h}z_{2}+z_{1}k_{3}k_{4}\right)\right]}{\Lambda_{h}\mu_{v}k_{1}k_{2}k_{3}k_{4}}\right],\\ z_{1}=\rho \left(1-\pi \right)k_{2}+\left(1-\left(1-\pi \right)\rho \right)k_{1},\\ z_{2}=\left(\alpha +\gamma_{s}\right)\left(1-\pi \right)\rho k_{2}+\left(\sigma_{r}+\gamma_{r}\right)\left(1-\left(1-\pi \right)\rho \right)k_{1}. \end{array}$$

**Proof**

Let us choose the rate of transmission of infection from an infectious mosquito to a susceptible human with *β*_*h*_ as the bifurcation parameter. We observe that *R*_0_ = 1  is equivalent to

(80) $$\begin{array}{c} \beta_{h}=\beta_{h}^{*}=\frac{\Lambda_{h}\mu_{v}k_{1}k_{2}k_{5}}{\phi^{2}\omega^{2}\beta_{v}\mu_{h}\Lambda_{v}\left(k_{2}\rho \left(1-\pi \right)+k_{1}\left(1-\left(1-\pi \right)\rho \right)\right)}, \end{array}$$

and the linearized Jacobian matrix evaluated at  *F*_0_  and *β*_*h*_^∗^ is denoted and given by

(81) $$\begin{array}{c} J\left(F_{0},\beta_{h}^{*}\right)=\left[\begin{array}{ccccccc} -\mu_{h} & 0 & 0 & \varepsilon & \theta & 0 & -k_{17}^{*}\\ 0 & -k_{1} & 0 & 0 & 0 & 0 & k_{27}^{*}\\ 0 & 0 & -k_{2} & 0 & 0 & 0 & k_{37}^{*}\\ 0 & \alpha & \sigma_{r} & -k_{3} & 0 & 0 & 0\\ 0 & \gamma_{s} & \gamma_{r} & 0 & -k_{4} & 0 & 0\\ 0 & -k_{62} & -k_{63} & 0 & 0 & -\mu_{v} & 0\\ 0 & k_{72} & k_{73} & 0 & 0 & 0 & -k_{5} \end{array}\right]. \end{array}$$

Here, *K*_17_^∗^ = *ϕωβ*_*h*_^∗^, *k*_27_^∗^ = (1 − *π*)*ρϕωβ*_*h*_^∗^, and *k*_37_^∗^ = (1 − (1 − *π*)*ρ*)*ϕωβ*_*h*_^∗^.

Now, the eigenvalues of $J\left(\begin{array}{cc} F_{0}, & \beta_{h}^{*} \end{array}\right)$ are the solutions of the characteristic equation $\text{ Det}\left[\;J\left(\begin{array}{cc} F_{0}, & \beta_{h}^{*} \end{array}\right)-\lambda I\right]=0$. Thus, the determinant is given by

(82) $$\begin{array}{c} \left|\begin{array}{ccccccc} -\mu_{h}-\lambda & 0 & 0 & \varepsilon & \theta & 0 & -k_{17}^{*}\\ 0 & -k_{1}-\lambda & 0 & 0 & 0 & 0 & k_{27}^{*}\\ 0 & 0 & -k_{2}-\lambda & 0 & 0 & 0 & k_{37}^{*}\\ 0 & \alpha & \sigma_{r} & -k_{3}-\lambda & 0 & 0 & 0\\ 0 & \gamma_{s} & \gamma_{r} & 0 & -k_{4}-\lambda & 0 & 0\\ 0 & -k_{62} & -k_{63} & 0 & 0 & -\mu_{v}-\lambda & 0\\ 0 & k_{72} & k_{73} & 0 & 0 & 0 & -k_{5}-\lambda \end{array}\right|=0. \end{array}$$

If and only if *λ*_1_ = −*μ*_*h*_ < 0,  *λ*_2_ = −*μ*_*v*_ < 0,  *λ*_3_ = −*k*_2_ < 0, and *λ*_4_ = −*k*_4_ < 0,

(83) $$\begin{array}{c} c_{0}\lambda^{3}+c_{1}\lambda^{2}+c_{2}\lambda +c_{3}=0, \end{array}$$

where

(84) $$\begin{array}{c} c_{0}=1,\\ c_{1}=k_{1}+k_{2}+k_{5},\\ c_{2}=k_{2}k_{5}+k_{1}\left(k_{2}+k_{5}\right)-\frac{\phi^{2}\omega^{2}\beta_{h}^{*}\beta_{v}\Lambda_{v}\mu_{h}}{\Lambda_{h}\mu_{v}},\\ c_{3}=k_{1}k_{2}k_{5}\left(1-R_{0}^{2}\right). \end{array}$$

If we substitute 1 (one) for  *R*_0_ into equation (83) or (84), then system (12) will have a simple zero eigenvalue, and the other eigenvalues have negative real parts. Therefore, the disease-free equilibrium point  *F*_0_ is nonhyperbolic.

Let us make the following change of state variables  *S*_*h*_ = *x*_1_, *I*_*hs*_ = *x*_2_, *I*_*hr*_ = *x*_3_, *T*_*h*_ = *x*_4_, *R*_*h*_ = *x*_5_, *S*_*v*_ = *x*_6_, and *I*_*v*_ = *x*_7_ using the vector notation $x={\left(\;\begin{array}{cc} x_{1}, & \begin{array}{ccc} x_{2},x_{3}, & x_{4}, & \begin{array}{ccc} x_{5}, & x_{6}, & x_{7} \end{array} \end{array} \end{array}\right)}^{T}$. System (12) can then be written in the form *dx*/*dt* = *F*(*x*); here, $F={\left(\;\begin{array}{cc} f_{1}, & \begin{array}{ccc} f_{2},f_{3}, & f_{4}, & \begin{array}{ccc} f_{5}, & f_{6}, & f_{7} \end{array} \end{array} \end{array}\right)}^{T}$ as shown below:

(85) $$\begin{array}{c} \left\{\begin{array}{c} \frac{dx_{1}}{dt}=f_{1}=\Lambda_{h}+\varepsilon x_{4}+\theta x_{5}-\left(\phi \omega \beta_{h}^{*}\frac{x_{7}}{x_{1}+x_{2}+x_{3}+x_{4}+x_{5}}+\mu_{h}\right)x_{1},\\ \frac{dx_{2}}{dt}=f_{2}=\rho \left(1-\pi \right)\phi \omega \beta_{h}^{*}\left(\frac{x_{7}}{x_{1}+x_{2}+x_{3}+x_{4}+x_{5}}\right)x_{1}-\left(\mu_{h}+\delta_{h}+\alpha +\gamma_{s}\right)x_{2},\\ \frac{dx_{3}}{dt}=f_{3}=\left(1-\left(1-\pi \right)\rho \right)\phi \omega \beta_{h}^{*}\left(\frac{x_{7}}{x_{1}+x_{2}+x_{3}+x_{4}+x_{5}}\right)x_{1}-\left(\mu_{h}+\delta_{h}+\gamma_{r}+\sigma_{r}\right)x_{3},\\ \frac{dT_{h}}{dt}=f_{4}=\alpha x_{2}+\sigma x_{3}-\left(\delta_{h}+\mu_{h}+\varepsilon \right)x_{4},\\ \frac{dx_{5}}{dt}=f_{5}=\gamma_{s}x_{2}+\gamma_{r}x_{3}-\left(\theta +\mu_{h}\right)x_{5},\\ \frac{dx_{6}}{dt}=f_{6}=\Lambda_{v}-\left(\phi \omega \beta_{v}\frac{x_{2}+x_{3}}{x_{1}+x_{2}+x_{3}+x_{4}+x_{5}}+\mu_{v}\right)x_{6},\\ \frac{dx_{7}}{dt}=f_{7}=\left(\phi \omega \beta_{v}\frac{x_{2}+x_{3}}{x_{1}+x_{2}+x_{3}+x_{4}+x_{5}}\right)x_{6}-\left(\mu_{v}+\delta_{v}\right)x_{7}, \end{array}\right. \end{array}$$

The coefficients *a* and *b* are defined in Theorem Appendix B.1. of [21]. That is,

(86) $$\begin{array}{c} a=\frac{1}{2}\overset{n}{\underset{k,i,j=1}{\sum }}v_{k}w_{i}w_{j}\frac{\partial^{2}f_{k}}{\partial x_{i}ðx_{j}}\left(S_{h}^{0},0,0,0,S_{v}^{0},0\;\right),\\ b=\overset{n}{\underset{k,i=1}{\sum }}v_{k}w_{i}\frac{\partial^{2}f_{k}}{\partial x_{i}ð\beta_{h}^{*}}\left(S_{h}^{0},0,0,0,S_{v}^{0},0\right). \end{array}$$

To compute the coefficient equations *a* and *b*, we determine the right and left eigenvectors corresponding to the zero eigenvalue. Thus, the components of the right eigenvectors denoted by  *w*_*i*_, for *i* = 1, ⋯, 7, are given by

(87) $$\begin{array}{c} \left[\begin{array}{ccccccc} -\mu_{h} & 0 & 0 & \varepsilon & \theta & 0 & -k_{17}^{*}\\ 0 & -k_{1} & 0 & 0 & 0 & 0 & k_{27}^{*}\\ 0 & 0 & -k_{2} & 0 & 0 & 0 & k_{37}^{*}\\ 0 & \alpha & \sigma_{r} & -k_{3} & 0 & 0 & 0\\ 0 & \gamma_{s} & \gamma_{r} & 0 & -k_{4} & 0 & 0\\ 0 & -k_{62} & -k_{63} & 0 & 0 & -\mu_{v} & 0\\ 0 & k_{72} & k_{73} & 0 & 0 & 0 & -k_{5} \end{array}\right]\left[\begin{array}{c} \;w_{1}\\ \;w_{2}\\ \;w_{3}\\ \;w_{4}\\ \;w_{5}\\ \;w_{6}\\ \;w_{7} \end{array}\right]=\left[\begin{array}{c} 0\\ 0\\ 0\\ 0\\ 0\\ 0\\ 0 \end{array}\right]. \end{array}$$

Equation (87) can be written as

(88) $$\begin{array}{c} \left\{\begin{array}{c} -\mu_{h}w_{1}+\varepsilon w_{4}+\theta w_{5}-k_{17}^{*}w_{7}=0,\\ -k_{1}w_{2}+k_{27}^{*}w_{7}=0,-k_{2}w_{3}+k_{37}^{*}w_{7}=0,\\ \alpha w_{2}+\sigma w_{3}-k_{3}w_{4}=0,\\ \gamma_{s}w_{2}+\gamma_{r}w_{3}-k_{4}w_{5}=0,\\ -k_{62}\left(w_{2}+w_{3}\right)-\mu_{\text{v}}w_{6}=0,\\ k_{72}\left(w_{2}+w_{3}\right)-k_{5}w_{7}=0. \end{array}\right. \end{array}$$

Solving equation (88) gives

(89) $$\begin{array}{c} w_{1}=\frac{\phi \omega \beta_{h}^{*}\left[\varepsilon k_{4}\left[\left(1-\pi \right)\rho \alpha k_{2}+\left(1-\left(1-\pi \right)\rho \right){\gamma \sigma }_{r}k_{1}\right]+\theta k_{3}\left[\rho \left(1-\pi \right)\gamma_{s}k_{2}+\left(1-\left(1-\pi \right)\rho \right)\gamma_{r}k_{1}\right]-k_{1}k_{2}k_{4}\right]}{\mu_{h}k_{1}k_{2}k_{3}k_{4}}w_{7},\\ w_{2}=\frac{k_{27}^{*}}{k_{1}}w_{7},\\ w_{3}=\frac{k_{37}^{*}}{k_{2}}w_{7},\\ w_{4}=\frac{\phi \omega \beta_{h}^{*}\left[\rho \left(1-\pi \right)\alpha k_{2}+\left(1-\left(1-\pi \right)\rho \right)\sigma_{r}k_{1}\right]}{k_{1}k_{2}k_{3}}w_{7},\\ w_{5}=\frac{\phi \omega \beta_{h}^{*}\left(\rho \left(1-\pi \right)\gamma_{s}k_{2}+\left(1-\left(1-\pi \right)\rho \right)\gamma_{r}k_{1}\right)}{k_{1}k_{2}k_{4}}w_{7},\\ w_{6}=-\frac{k_{5}}{\mu_{v}}w_{7}. \end{array}$$

Further, here,  *w*_7_  is a positive quantity, i.e., *w*_7_ > 0.

Similarly, the components of the left eigenvector denoted by *v*_*i*_, for  *i* = 1, ⋯, 7, are given by

(90) $$\begin{array}{c} {\left[\begin{array}{ccccccc} -\mu_{h} & 0 & 0 & \varepsilon & \theta & 0 & -k_{17}^{*}\\ 0 & -k_{1} & 0 & 0 & 0 & 0 & k_{27}^{*}\\ 0 & 0 & -k_{2} & 0 & 0 & 0 & k_{37}^{*}\\ 0 & \alpha & \sigma_{r} & -k_{3} & 0 & 0 & 0\\ 0 & \gamma_{s} & \gamma_{r} & 0 & -k_{4} & 0 & 0\\ 0 & -k_{62} & -k_{63} & 0 & 0 & -\mu_{v} & 0\\ 0 & k_{72} & k_{73} & 0 & 0 & 0 & -k_{5} \end{array}\right]}^{T}\left[\begin{array}{c} \;v_{1}\\ \;v_{2}\\ \;v_{3}\\ \;v_{4}\\ \;v_{5}\\ \;v_{6}\\ \;v_{7} \end{array}\right]=\left[\begin{array}{c} 0\\ 0\\ 0\\ 0\\ 0\\ 0\\ 0 \end{array}\right]. \end{array}$$

Equation (90) can be written as

(91) $$\begin{array}{c} \left\{\begin{array}{c} -\mu_{h}v_{1}=0\\ -k_{1}v_{2}+\alpha v_{4}+\gamma_{s}v_{5}-k_{62}\left(\;v_{6}-v_{7}\right)=0\\ -k_{2}v_{3}+\sigma_{r}v_{4}+\gamma_{s}v_{5}-k_{63}\left(\;v_{6}-v_{7}\right)=0\\ \;{\varepsilon v}_{1}-k_{3}v_{4}=0\\ \theta v_{1}-k_{4}v_{5}=0\\ -\mu_{\text{v}}v_{6}=0\\ -k_{17}^{*}v_{1}+l_{27}^{*}v_{2}+k_{37}^{*}v_{3}-k_{5}v_{7}=0 \end{array}\right. \end{array}$$

Solving equation (91) gives

(92) $$\begin{array}{c} v_{1}=v_{4}=v_{5}=v_{6}=0,\\ v_{2}=\frac{k_{62}}{k_{1}}v_{7},\\ v_{3}=\frac{k_{62}}{k_{2}}v_{7}\\ v_{7}=v_{7}>0. \end{array}$$

Taking into account system (85) and considering only the nonzero components of the left eigenvector *v*, it follows that the *f*_is_ denotes the right-hand side of system (85). It can be checked that

(93) $$\begin{array}{c} \frac{\partial^{2}f_{2}}{\partial x_{7}\partial x_{2}}\left(F_{0}\right)=\frac{\partial^{2}f_{2}}{\partial x_{7}\partial x_{3}}\left(F_{0}\right)=\frac{\partial^{2}f_{2}}{\partial x_{7}\partial x_{4}}\left(F_{0}\right)=\frac{\partial^{2}f_{2}}{\partial x_{7}\partial x_{5}}\left(F_{0}\right)=-\frac{\rho \left(1-\pi \right)\phi \omega \beta_{h}^{*}}{S_{h}^{0}},\\ \frac{\partial^{2}f_{3}}{\partial x_{7}\partial x_{2}}\left(F_{0}\right)=\frac{\partial^{2}f_{3}}{\partial x_{7}\partial I_{3}}\left(F_{0}\right)=\frac{\partial^{2}f_{3}}{\partial x_{7}\partial x_{3}}\left(F_{0}\right)=\frac{\partial^{2}f_{3}}{\partial x_{7}\partial x_{5}}\left(F_{0}\right)=-\frac{\left(1-\left(1-\pi \right)\rho \right)\phi \omega \beta_{h}^{*}}{S_{h}^{0}},\\ \frac{\partial^{2}f_{7}}{\partial {Ix}_{2}\partial {Sx}_{1}}\left(F_{0}\right)=\frac{\partial^{2}f_{7}}{\partial {Ix}_{2}\partial x_{4}}\left(F_{0}\right)=\frac{\partial^{2}f_{7}}{\partial {Ix}_{2}\partial {Rx}_{5}}\left(F_{0}\right)=\frac{\partial^{2}f_{7}}{\partial x_{3}\partial {Sx}_{1}}\left(F_{0}\right)=\frac{\partial^{2}f_{7}}{\partial x_{3}\partial x_{4}}\left(F_{0}\right)=\frac{\partial^{2}f_{7}}{\partial I_{3}\partial x_{5}}\left(F_{0}\right)=-\frac{\phi \omega \beta_{v}S_{v}^{0}}{{\left(S_{h}^{0}\right)}^{2}},\\ \frac{\partial^{2}f_{7}}{\partial x_{2}^{2}}\left(F_{0}\right)=\frac{\partial^{2}f_{7}}{\partial {\text{x}}_{h}^{2}}\left(F_{0}\right)=\frac{\partial^{2}f_{7}}{\partial x_{2}\partial x_{3}}=-\frac{2{\phi \omega \beta }_{v}S_{v}^{0}}{{\left(S_{h}^{0}\right)}^{2}},\\ \frac{\partial^{2}f_{7}}{\partial x_{2}\partial x_{6}}\left(x_{0},0\right)=\frac{\partial^{2}f_{7}}{\partial x_{3}\partial x_{6}}\left(x_{0},0\right)=\frac{\phi \omega \beta_{v}}{S_{h}^{0}},\\ \frac{\partial^{2}f_{2}}{\partial x_{7}\partial \beta_{h}^{*}}\left(x_{0},0\right)=\phi \omega \rho \left(1-\pi \right),\\ \frac{\partial^{2}f_{3}}{\partial x_{7}\partial \beta_{h}^{*}}\left(x_{0},0\right)=\phi \omega \left(1-\left(1-\pi \right)\rho \right). \end{array}$$

Now, using the nonzero components of left eigenvector  *v*, right eigenvector *w*, and the nonzero partial derivatives ((*∂*^2^*f*_*k*_)/(*∂x*_*i*_*∂x*_*j*_) (*F*_0_)), ((*∂*^2^*f*_*k*_)/(*∂x*_*i*_*∂β*_*h*_^∗^) (*∂*^2^*f*_k_/*∂x*_*i*_*∂β*_*h*_^∗^)(*F*_0_)), the coefficients *a* and *b*  are determined as

(94) $$\begin{array}{c} a=\left(\frac{\phi^{2}\omega^{2}\mu_{h}\beta_{h}^{*}\beta_{v}}{\Lambda_{h}\left(\mu_{h}+\delta_{h}+\alpha +\gamma_{s}\right)}\right){\text{B}}_{0}v_{7}w_{7}^{2},\\ b=\frac{v_{7}^{2}w_{7}\phi^{2}\omega^{2}\beta_{v}\mu_{h}\Lambda_{v}\left(\left(1-\pi \right)\rho k_{2}+\left(1-\left(1-\pi \right)\rho \right)k_{1}\right)}{\Lambda_{h}\mu_{v}k_{1}k_{2}}. \end{array}$$

Here, *B*_0_  denotes the following parametric expression:

(95) $$\begin{array}{c} B_{0}=\frac{a\phi \omega \beta_{v}\Lambda_{v}}{\mu_{v}\Lambda_{h}k_{2}}-\left[\frac{a\Lambda_{h}k_{1}k_{3}k_{4}k_{5}+\Lambda_{v}\phi \omega \beta_{v}\left[{\left(1-\pi \right)}^{2}\rho^{2}k_{2}^{2}k_{3}k_{4}+a\left(\varepsilon +\theta +2\mu_{h}b+{ak}_{3}k_{4}\right)\right]}{\Lambda_{h}\mu_{v}k_{1}k_{2}k_{3}k_{4}}\right].\\ a=\rho \left(1-\pi \right)k_{2}+\left(1-\left(1-\pi \right)\rho \right)k_{1},\\ b=\left(\alpha +\gamma_{s}\right)\left(1-\pi \right)\rho k_{2}+\left(\sigma_{r}+\gamma_{r}\right)\left(1-\left(1-\pi \right)\rho \right)k_{1}. \end{array}$$

Clearly, it can be observed that *b*  is absolutely a positive quantity while *a* is negative if *B*_0_ < 0. Hence, it is a forward bifurcation.

Therefore, we conclude that the model equations in (12) exhibit forward bifurcation at *R*_0_ = 1 if the condition *B*_0_ < 0  is satisfied.

### 3.9. Local Stability of Endemic Equilibrium

**Theorem 7 .**

The endemic equilibrium point (*E*^∗^) of system (12) is locally asymptotically stable if *R*_0_ > 1.

**Proof**

The Jacobian matrix of system (12) evaluated at  *E*^∗^ is given by

(96) $$\begin{array}{c} J\left(E^{*}\right)=\left[\begin{array}{ccccccc} -P & 0 & 0 & \varepsilon & \theta & 0 & -Q\\ R & -k_{1} & 0 & 0 & 0 & 0 & S\\ T & 0 & -k_{2} & 0 & 0 & 0 & Z\\ 0 & \alpha & \sigma_{r} & -k_{3} & 0 & 0 & 0\\ 0 & \gamma_{s} & \gamma_{r} & 0 & -k_{4} & 0 & 0\\ 0 & -X & -X & 0 & 0 & -Y & 0\\ 0 & X & X & 0 & 0 & 0 & -k_{5} \end{array}\right],\\ P=\omega \phi \beta_{h}\frac{I_{v}^{*}}{N_{h}^{*}}+\mu_{h},\\ R=\rho \left(1-\pi \right)\omega \phi \beta_{h}\frac{I_{v}^{*}}{N_{h}^{*}},\\ T=\left(1-\left(1-\pi \right)\;\rho \right)\omega \phi \beta_{h}\frac{I_{v}^{*}}{N_{h}^{*}},\\ Q=\omega \phi \beta_{h}\frac{S_{h}^{*}}{N_{h}^{*}},\\ S=\rho \left(1-\pi \right)\omega \phi \beta_{h}\frac{S_{h}^{*}}{N_{h}^{*}},\\ Z=\left(1-\left(1-\pi \right)\;\rho \right)\omega \phi \beta_{h}\frac{S_{h}^{*}}{N_{h}^{*}},\\ X=\omega \phi \beta_{v}\frac{S_{v}^{*}}{N_{h}^{*}}\left(1-\frac{\left(I_{\text{hs}}^{*}+I_{\text{hr}}^{*}\right)}{N_{h}^{*}}\;\right),\\ Y=\omega \phi \beta_{v}\frac{\left(I_{\text{hs}}^{*}+I_{\text{hr}}^{*}\right)}{N_{h}^{*}}+\mu_{v}. \end{array}$$

The eigenvalues of the *J*(*E*^∗^) are given by clearly *λ*_1_ = −(*ωϕβ*_*v*_((*I*_hs_^∗^ + *I*_hr_^∗^)/*N*_*h*_^∗^) + *μ*_*v*_ ) < 0, and its associate characteristic equation is

(97) $$\begin{array}{c} \lambda^{6}+e_{1}\lambda^{3}+e_{2}\lambda^{2}+e_{3}\lambda^{3}+e_{4}\lambda^{2}+e\lambda +e_{6}=0. \end{array}$$

Here,

(98) $$\begin{array}{c} \left\{\begin{array}{c} e_{1}=P+k_{1}+k_{2}+k_{3}+k_{4}+k_{5},\\ e_{2}=k_{3}k_{4}+\left(k_{3}+k_{4}\right)\left(P+k_{1}+k_{2}+k_{5}\right)+\left(P+k_{1}\right)\left(k_{2}+k_{5}\right)+k_{2}k_{5}-XU,\\ e_{3}=k_{3}k_{4}+\left(k_{2}+k_{5}\right)\left(k_{3}k_{4}+\left(P+k_{1}\right)\left(k_{3}+k_{4}\right)+Pk_{1}\right)+Pk_{1}\left(k_{3}+k_{4}\right)+\left(k_{2}k_{5}-XZ\right)\left(P+k_{1}+k_{3}+k_{4}\right),\\ e_{4}=k_{3}k_{4}\left(Pk_{1}+k_{2}+k_{5}+k_{2}k_{5}-XU\right)+\left(k_{3}+k_{4}\right)\left(Pk_{1}+\left(k_{2}+k_{5}\right)Pk_{1}+Pk_{1}\left(k_{2}k_{5}-XZ\right)\right)+\\ Pk_{1}\left(k_{2}k_{5}-XZ\right)+\theta \gamma_{s}R\left(1+k_{2}\right)+\theta \gamma_{s}T\left(1+k_{1}\right)+\left(k_{3}+k_{5}\right)\theta \left(\gamma_{s}R+\gamma_{s}T\right)+\varepsilon T\sigma_{r}\left(k_{1}+k_{4}+k_{5}\right)+\\ Q\left(\gamma_{s}Tk_{1}+\gamma_{r}Rk_{2}\;\right)+Q\left(k_{3}+k_{5}\right)\left(\gamma_{s}T+\gamma_{r}R\right),\\ e_{5}=\left(k_{2}+k_{5}\right)Pk_{1}k_{3}k_{4}+k_{3}k_{4}\left(k_{2}k_{5}-XZ\right)+\left(k_{3}+k_{4}\right)Pk_{1}\left(k_{2}k_{5}-XZ\right)+\\ \;\varepsilon T\sigma_{r}\left(k_{1}k_{5}+k_{4}\left(k_{1}+k_{5}\right)\right)+\varepsilon X\left(\sigma_{r}-\alpha \right)\left(RZ-ST\right)+\theta k_{3}k_{5}\left(\gamma_{r}T+\gamma_{s}R\right)+\theta \left({\text{k}}_{3}+k_{5}\right)\left(\gamma_{r}Tk_{1}-\gamma_{s}Rk_{2}\right)+\\ Q\left(\gamma_{s}Tk_{1}+\gamma_{r}Rk_{2}\right)+\theta X\left(\gamma_{s}-\gamma_{r}\right)\left(RZ-ST\right)+Q\left(RZX\left(\left(\gamma_{s}-\gamma_{r}\right)\right)+\left(\gamma_{r}T-\gamma_{s}R\right)\right)k_{2}k_{5},\\ e_{6}=Pk_{1}m_{2}k_{3}k_{4}k_{5}+\varepsilon k_{4}\left(T\sigma_{r}+k_{1}k_{5}+X\left(RZ-ST\right)\right)\left(\sigma_{r}-\alpha \right)+\theta k_{3}k_{5}\left(\gamma_{r}T+\gamma_{s}R\right)+\\ \left(k_{3}+k_{5}\right)\left(\theta \left(\gamma_{s}Tk_{1}+\gamma_{r}Rk_{2}\right)+Q\left(\gamma_{s}Tk_{1}-\gamma_{r}Rk_{2}\right)\right)+X\left(\gamma_{s}-\gamma_{\text{r}}\right)\left(\theta \left(RZk_{5}-STk_{3}\right)+QRZk_{5}\right). \end{array}\;\right. \end{array}$$

The Routh-Hurwitz criteria for polynomial equation (97) will give six negative eigenvalues if the conditions given below are satisfied: *e*_*i*_ > 0, for *i* = 1, 2, 3, ⋯, 6. The relevant Routh-Hurwitz criteria in [19, 25] could be used to show that model system (12) is locally asymptotically stable when *R*_0_ > 1.

## 4. Extension of the Model into an Optimal Control

### 4.1. Optimization Process

For malaria, control efforts are carried out to limit the spread of the disease and free the community from the burden of the disease. Optimal control theory is a method that has been widely used to solve for an extremum value of an objective function involving dynamic variables. In this section, optimal control theory of [26] has been applied in deriving optimal control problem that incorporates the time-dependent control measures, namely, prevention of drug resistance, insecticide-treated bed net (ITN), treatment, and indoor residual spray (IRS) as functions of time to investigate the optimal control efforts needed to control malaria disease. The controls are assigned reasonable upper and lower bounds and practiced on time interval [*t*_0_, *t*_*f*_], where *t*_0_ and *t*_f_ are the initial and final time, respectively. The control variables as used in the basic malaria model (12) are described as follows:

The preventive control measure drug resistance at time *t* is denoted by  *u*_1_; this is aimed at minimizing the proportion of the emergence of drug resistance of malaria strains as well as spread of the disease dynamics. It can be implemented by improving the way drugs are used through improving prescribing, follow-up practices, and patient compliance.

The preventive control measure insecticide-treated bed net (ITN) at time *t* is denoted by  *u*_2_; it has twofold effects on the malaria disease dynamics: (i) reduces the number of bites from mosquitoes as they physically provide a barrier between the infectious mosquitoes and (ii) reduces the population of the mosquitoes by killing them after they land on the treated net.

The control measure treatment with drugs at time *t* is denoted by  *u*_3_; this includes treating individuals who developed symptoms of the disease.

The preventive control measure indoor residual spray (IRS) at time *t* is denoted by  *u*_4_  as preventive measure; i.e., insecticide spray on the breeding site of mosquitoes reduces the number of mosquito populations by killing the rest indoors after feeding.

After incorporating the above controls into basic model system (12), we get the following modified state equation:

(99) $$\begin{array}{c} \left\{\begin{array}{c} \frac{dS_{h}}{dt}=\Lambda_{h}+\left(\varepsilon +u_{1}+\left(1-\tau u_{3}\right)\right)T_{h}+\theta R_{h}-\left(\left(1-u_{2}\right)\lambda_{h}+\mu_{h}\right)S_{h},\\ \frac{dI_{hs}}{dt}=\left(1-u_{2}\right)\rho \left(1-\left(1-u_{1}\right)\pi \right)\lambda_{h}S_{h}-\left(\mu_{h}+\delta_{h}+\alpha +\left(\gamma_{s}+\tau u_{3}\right)\right)I_{hs},\\ \frac{dI_{hr}}{dt}=\left(1-u_{2}\right)\left(1-\left(1-\left(1-u_{1}\right)\pi \right)\rho \right)\lambda_{h}S_{h}-\left(\mu_{h}+\delta_{h}+\sigma_{r}+\gamma_{r}\right)I_{hr},\\ \frac{dT_{h}}{dt}=\alpha I_{hs}+\sigma I_{hr}-\left(\delta_{h}+\mu_{h}+\varepsilon +u_{1}+\left(1-\tau u_{3}\right)\right)T_{h},\\ \frac{dR_{h}}{dt}=\left(\gamma_{s}+\tau u_{3}\right)I_{hs}+\gamma_{r}I_{hr}-\left(\theta +\mu_{h}\right)R_{h},\\ \frac{dS_{v}}{dt}=\Lambda_{v}-\left(\left(1-u_{2}\right)\lambda_{v}+\mu_{v}+\delta u_{2}+\beta u_{4}\right)S_{v},\\ \frac{dI_{v}}{dt}=\left(1-u_{2}\right)\lambda_{v}S_{v}-\left(\mu_{v}+\delta_{v}+\delta u_{2}+\beta u_{4}\right)I_{v}. \end{array}\;\right. \end{array}$$

Here, we also use following the approach developed by [26] and proposed the following objective function *J* which is used to minimize the number of infected humans with drug-sensitive and drug-resistant malaria parasite strains, infective in treated human populations, and total mosquito populations while keeping the costs of applying the controls  *u*_1_,  *u*_2_,  *u*_3_, and  *u*_4_  as low as possible.

(100) $$\begin{array}{c} J=\min\int_{0}^{t_{f}}\left(A_{1}I_{\text{hs}}+A_{2}I_{\text{hr}}+A_{3}T_{h}+A_{4}I_{v}+\frac{1}{2}\overset{4}{\underset{1}{\sum }}d_{i}u_{i}^{2}\right)dt, \end{array}$$

where *i* = 1, 2, 3, 4 and *A*_1_, *A*_2_, *A*_3_, and *A*_4_  and *d*_1_,  *d*_2_,  *d*_3_, and,  *d*_4_ are the coefficients associated to the state variable and controls, respectively. Following the approach of [26], the cost of the controls has been chosen to be quadratic.

Thus, the goal is to find an optimal control quadruple, *u*_1_^∗^, *u*_2_^∗^,  *u*_3_^∗^, and  *u*_4_^∗^ such that

(101) $$\begin{array}{c} J\left(\;u_{1}^{*},u_{2}^{*},u_{3}^{*},u_{4}^{*}\right)=\min\left\{J\left(\;u_{1},u_{2},u_{3},u_{4}\right)\text{: }u_{1},u_{2},u_{3},u_{4}\epsilon U\right\}, \end{array}$$

where $U=\left\{\begin{array}{ccccc} u_{1}\left(t\right) & u_{2}\left(t\right) & u_{3}\left(t\right) & u_{4}\left(t\right) & :0\leq u_{i}<1,i=1,2,\cdots ,4,0\leq t\leq t_{f} \end{array}\right\}$ is the control set.

Pontryagin's maximum principle [27] converts system (99) with (100) and (101) into a problem of minimizing pointwise the Hamiltonian *H* with respect to  *u*_1_,  *u*_2_,  *u*_3_, and  *u*_4_. Thus, the Hamiltonian *H* equation is given by

(102) $$\begin{array}{c} H=\left(S_{h},I_{\text{hs}},I_{\text{hr}},T_{h},R_{h},S_{v}\;I_{v},t\right)=L\left(I_{\text{hs}},I_{\text{hr}},T_{h},I_{v},u_{1},u_{2},u_{3},u_{4},t\right)+\lambda_{1}\frac{dS_{h}}{dt}+\lambda_{2}\frac{dI_{\text{hs}}}{dt}+\lambda_{3}\frac{dI_{\text{hr}}}{dt}+\lambda_{4}\frac{dT_{h}}{dt}+\lambda_{5}\frac{dR_{h}}{dt}+\lambda_{6}\frac{dS_{v}}{dt}+\lambda_{7}\frac{dI_{v}}{dt}. \end{array}$$

Here, *L*(*I*_hs_, *I*_hr_, *T*_*h*_, *I*_*v*_, *u*_1_, *u*_2_, *u*_3_, *u*_4_, *t*) = *A*_1_*I*_hs_ + *A*_2_*I*_hr_ + *A*_3_*T*_*h*_ + *A*_4_*I*_*v*_ + 1/2∑_1_^4^*d*_*i*_*u*_*i*_^2^ for *i* = 1, 2, 3, 4 and *λ*_*i*_, for *i* = 1, 2, 3, 4, 5, 6, 7, are adjoint variable. Using the existence result for the optimal control [28, 29], we established the following theorem as follows.

**Theorem 8 .**

There exists a set of an optimal control $\;u_{i}^{*}=\left(\;u_{1}^{*},u_{2}^{*},\begin{array}{cc} \;u_{3,}^{*} & \;u_{4}^{*} \end{array}\right)\;$ and corresponding state solution,  *S*_*h*_^∗∗^, *I*_*hs*_^∗∗^, *I*_*hr*_^∗∗^, *T*_*h*_^∗∗^, *R*_*h*_^∗∗^,  *S*_*v*_^∗∗^, and *I*_*v*_^∗∗^, that minimizes $J\left(u_{1},u_{2},\begin{array}{cc} u_{3}, & u_{4} \end{array}\right)$ over *U*  subject to (99). Further, there exist adjoint functions *λ*_1_(*t*), ⋯,  *λ*_7_(*t*) and *u*_1_(*t*), ⋯*u*_4_(*t*) satisfying

(103) $$\begin{array}{c} \left\{\begin{array}{c} \;\frac{d\lambda_{1}}{dt}=\mu_{h}\lambda_{1}+\left(1-u_{2}\right)\lambda_{h}\left(\lambda_{1}-\rho \left(1-\left(1-u_{1}\right)\pi \right)\lambda_{2}-\left(1-\left(1-\left(1-u_{1}\right)\pi \right)\rho \right)\lambda_{3}\right)+\frac{\left(1-u_{2}\right)S_{v}\;}{N_{h}}\lambda_{v}\left(\lambda_{7}-\lambda_{6}\right),\\ \frac{d\lambda_{2}}{dt}=-A_{1}+\alpha \left(\lambda_{2}-\lambda_{4}\right)-\left(\gamma_{s}+\tau u_{3}\right)\left(\lambda_{2}-\lambda_{5}\right)+\left(\mu_{h}+\delta_{h}\right)\lambda_{2}+\frac{\left(1-u_{2}\right)\phi \omega \beta_{v}S_{v}\;}{N_{h}}\left(1-\frac{I_{hs}+I_{hr}}{N_{h}}\right)\left(\lambda_{6}-\lambda_{7}\right),\\ \;\\ \frac{d\lambda_{3}}{dt}=-A_{2}+\sigma_{r}\left(\lambda_{3}-\lambda_{4}\right)-\gamma_{r}\left(\lambda_{3}-\lambda_{5}\right)+\left(\mu_{h}+\delta_{h}\right)\lambda_{2}\frac{\left(1-u_{2}\right)\phi \omega \beta_{v}S_{v}\;}{N_{h}}\left(1-\frac{I_{hs}+I_{hr}}{N_{h}}\right)\left(\lambda_{6}-\lambda_{7}\right),\\ \frac{d\lambda_{4}}{dt}=-A_{3}+\left(\varepsilon +u_{1}+\left(1-\tau u_{3}\right)\right)\left(\lambda_{4}-\lambda_{1}\right)+\left(\mu_{h}+\delta_{h}\right)\lambda_{4}+\frac{\left(1-u_{2}\right)S_{v}\;}{N_{h}}\lambda_{d}\left(\lambda_{7}-\lambda_{6}\right),\\ \frac{d\lambda_{5}}{dt}=\mu_{h}\lambda_{5}+\theta \left(\lambda_{5}-\lambda_{1}\right)+\frac{\left(1-u_{2}\right)S_{v}\;}{N_{h}}\lambda_{v}\left(\lambda_{7}-\lambda_{6}\right),\\ \;\frac{d\lambda_{6}}{dt}=\left(1-u_{2}\right)\lambda_{v}\left(\lambda_{6}-\lambda_{7}\right)+\left(\mu_{v}+\delta u_{2}+\beta u_{4}\right)\lambda_{6},\\ \frac{d\lambda_{7}}{dt}=\left(1-u_{2}\right)\frac{\phi \omega \beta_{h}S_{h}}{N_{h}}\left(\lambda_{1}-\rho \left(1-\left(1-u_{1}\right)\pi \right)\lambda_{2}-\left(1-\left(1-\left(1-u_{1}\right)\pi \right)\rho \right)\lambda_{3}\right)+\left(\mu_{v}+\delta_{v}+\delta u_{2}+\beta u_{4}\right)\lambda_{7}-A_{4}, \end{array}\;\right. \end{array}$$

with transversality conditions

(104) $$\begin{array}{c} \lambda_{i}\left(t_{f}\right)=0\text{ for }i=1,2,3,4,5,6,7. \end{array}$$

Further, the optimal controls  *u*_1_^∗^, *u*_2_^∗^, *u*_3_^∗^, and  *u*_4_^∗^ are given by

(105) $$\begin{array}{c} u_{1}^{*}=\min\left\{\max\left(0,\frac{\left(1-u_{2}\right)\pi \rho \lambda_{h}S_{h}\left(\lambda_{3}-\lambda_{2}\right)+\left(\lambda_{4}-\lambda_{1}\right)T_{h}}{d_{1}}\right),1\right\}, \end{array}$$

(106) $$\begin{array}{c} u_{2}^{*}=\min\left\{\max\left(0,\frac{\lambda_{h}S_{h}\left(\left(1-\left(1-u_{1}\right)\pi \right)\rho \lambda_{2}+\left(1-\left(1-\left(1-u_{1}\right)\pi \right)\rho \right)\lambda_{3}-\lambda_{1}\right)+\lambda_{v}S_{v}\left(\lambda_{7}-\lambda_{6}\right)+\delta \left(S_{v}\lambda_{6}+I_{v}\lambda_{7}\right)}{d_{2}}\right),1\right\}, \end{array}$$

(107) $$\begin{array}{c} u_{3}^{*}=\min\left\{\max\left(0,\frac{\tau \left(\lambda_{1}-\lambda_{4}\right)T_{h}+\tau \left(\lambda_{2}-\lambda_{5}\right)I_{\text{hs}}}{d_{3}}\right),1\right\}, \end{array}$$

(108) $$\begin{array}{c} u_{4}^{*}=\min\left\{\max\left(0,\frac{\beta \left({\text{S}}_{\text{v}}\lambda_{6}+{\text{I}}_{\text{v}}\lambda_{7}\right)}{d_{4}}\right),1\right\}. \end{array}$$

**Proof**

The existence of the optimal control follows from Fleming and Rishel [29] due to convexity of the integrand objective functional *J* in (100) with respect to *u*_*i*_, *i* = 1, 2, 3, 4 over the convex and closed control set *U*. System (99) satisfies Lipschitz property with respect to state variables since the state solutions are bounded. Differential equation (103) governing the adjoint variables *λ*_1_, *λ*_2_, ⋯, *λ*_7_ is obtained by partial differentiation of the Hamiltonian *H* in (102) with respect to the corresponding state variables, that is, (*dλ*_1_)/*dt* = −(*∂H*/*∂S*_*h*_),  (*dλ*_2_)/*dt* = −(*∂H*/*∂I*_hs_),  (*dλ*_3_)/*dt* = −(*∂H*/*∂I*_*hr*_),  (*dλ*_4_)/*dt* = −(*∂H*/*∂T*_*h*_), (*dλ*_5_)/*dt* = −(*∂H*/*∂R*_*h*_), *d*6/*dt* = −(*∂H*/*∂S*_*v*_), and (*dλ*_7_)/*dt* = −(*∂H*/*∂I*_*v*_) with terminal condition (104). The optimal control given by (105) is obtained by partial derivative of the Hamiltonian *H* in (102) with respect to each control  *u*_*i*_  and solving ( *∂H*)/(*∂*u_*i*_) = 0, for *i* = 1, 2, 3, 4.

## 5. Numerical Simulations and Cost-Effectiveness Analysis

### 5.1. Numerical Simulations

In this section, the optimality system, that is, state system (99) and adjoint system (103) with the optimal control given by (105), was solved numerically by applying Runge-Kutta fourth-order schemes of the approach [26]. The implementation of the scheme was done using the MATLAB package.

The parameter values provided in Table 1 are used so that *R*_0_ = 1.1937255489 > 1. The simulations of the model are done by using the initial conditions given by  *S*_*h*_(0) = 800, *I*_*hs*_(0) = 30, *I*_*hr*_(0) = 30, *T*_*h*_(0) = 30, *R*_*h*_(0) = 10, *S*_*v*_(0) = 5000, and *I*_*v*_(0) = 100. To minimize malaria infectious humans and the total mosquito populations as well as minimize the associated costs of controls, the weight constant values in objective function (100) are chosen so that  *A*_1_ = *A*_2_ = *A*_3_ = *A*_4_ = *d*_1_ = *d*_2_ = *d*_3_ = *d*_4_ = 4.

In order to estimate the impact of the incorporated time-dependent control measures on the malaria disease dynamics, we proposed four optimal combinations of control strategies. These strategies have been chosen based on their effectiveness in minimizing the spread of the malaria disease. To find the solution, we applied numerical methods, that is, systems (99) and (103) with (105) numerically solved by using the parameter values given in Table 1 and MATLAB software and applying Runge-Kutta fourth-order schemes. Thus, the proposed optimal combinations are as follows:

1. Strategy a: combination of the use of preventive control of drug resistance, insecticide-treated net (ITN), and treatment of infective individuals
2. Strategy b: combination of the use of preventive control of drug resistance, indoor residual spray (IRS) for vector control, and treatment of infective individuals
3. Strategy c: combination of the use of insecticide-treated nets ITN, indoor residual spray (IRS) for vector control, and treatment of infective individuals
4. Strategy d: combination of the use of preventive control of drug resistance, insecticide-treated nets ITN, indoor residual spray (IRS), and treatment of infective individuals

*Strategy a*: control with the prevention of drug resistance, insecticide-treated net (ITN), and treatment (*u*_1_ ≠ 0, *u*_2_ ≠ 0, *u*_3_ ≠ 0, and *u*_4_ = 0)

In this strategy, we compare the strategy a situation where no control (*u*_1_ = 0, *u*_2_ = 0, *u*_3_ = 0, and *u*_4_ = 0) was used with the application of strategy a. It can be seen from Figures 3(a)–3(f) that there is a significant increase in the number of susceptible and recovered human populations and a significant decrease in the number of infected with drug-sensitive strains, infected with drug-resistant strains, infective in treated human populations, and infected mosquito populations compared to the strategy with no control at a given time, respectively. From this, one can observe that strict application of strategy a for a period between 10 and 30 days is sufficient to reduce the number of individuals with malaria symptoms and malaria-infected vectors to zero. It can be noted that a combination of the prevention of drug resistance, insecticide-treated nets ITN, and treatment can play an important role in minimizing malaria infectious. The control profile shown in Figure 3(g) shows that controls  *u*_1_, *u*_2_, and  *u*_3_ decrease from the maximum of 100% to the lower bound. This suggests that a high effort is required for preventive control of drug resistance  *u*_1_, insecticide-treated net (ITN)  *u*_2_, and medical treatment  *u*_3_ of individuals under this strategy.

*Strategy b*: control with the prevention of drug resistance, indoor residual spray (IRS), and treatment (*u*_1_ ≠ 0, *u*_2_ = 0, *u*_3_ ≠ 0, and *u*_4_ ≠ 0)

In this strategy, we compare the strategy a situation where no control (*u*_1_ = 0, *u*_2_ = 0, *u*_3_ = 0, and *u*_4_ = 0) was used with the application of strategy b. It can be seen from Figures 4(a)–4(f) that there is a significant increase in the number of susceptible and recovered human populations and a significant decrease in the number of infected with drug-sensitive strains, infected with drug-resistant strains, infective in treated human populations, and infected mosquito populations compared to the strategy with no control at a given time, respectively. Even though this strategy minimizes the number of malaria infectious populations, however, it is not enough to eliminate the disease at a given time, and hence, there is a need for additional control effort to eliminate the disease out of the community. The control profile shown in Figure 4(g) shows that controls  *u*_1_, *u*_3_, and  *u*_4_ decrease from the maximum of 100% to the lower bound. This suggests that a high effort is required for preventive control of drug resistance  *u*_1_, indoor residual spray (IRS)  *u*_4_, and medical treatment  *u*_3_ of individuals under this strategy.

*Strategy c*: control with insecticide-treated net (ITN), indoor residual spray (IRS), and treatment (*u*_1_ = 0, *u*_3_ ≠ 0, *u*_3_ ≠ 0, and *u*_4_ ≠ 0)

In this strategy, we compare the strategy a situation where no control (*u*_1_ = 0, *u*_2_ = 0, *u*_3_ = 0, and *u*_4_ = 0) was used with the application of strategy c. It can be seen from Figures 5(a)–5(f) that there is a significant increase in the number of susceptible and recovered human populations and a dramatic decrease in the number of infected with drug-sensitive strains, infected with drug-resistant strains, infective in treated human populations, and infected mosquito populations compared to the strategy with no control at a given time, respectively. With the application of strategy d,  *I*_*v*_ within 8 days, *I*_*hs*_ within 10 days, *T*_*h*_ within 11 days, and  *I*_*hr*_  within 30 days will be eliminated from the system. This result is a bit more promising than strategy a and strategy b. The control profile shown in Figure 5(g) shows that control  *u*_3_ is at 55% initially and decreases from the maximum of 65% to the lower bound while controls *u*_2_ and  *u*_4_ decrease from the maximum of 100% to the lower bound within 90 days. This suggests that a high effort is required for the use of insecticide-treated net  *u*_2_ and indoor residual spray (IRS)  *u*_4_ for vector control, and there is a low effort for the use of medical treatment  *u*_3_ of individuals under this strategy.

*Strategy d*: control with the prevention of drug resistance, insecticide-treated net (ITN), indoor residual spray (IRS), and treatment (*u*_1_ ≠ 0, *u*_2_ ≠ 0, *u*_3_ ≠ 0, and *u*_4_ ≠ 0)

In this strategy, we compare the strategy a situation where no control (*u*_1_ = 0, *u*_2_ = 0, *u*_3_ = 0, and *u*_4_ = 0) was used with the application of strategy d. It can be seen from Figures 6(a)–6(f) that there is a significant increase in the number of susceptible and recovered human populations and a significant decrease in the number of infected with drug-sensitive strains, infected with drug-resistant strains, infective in treated human populations, and infected mosquito populations compared to the strategy with no control at a given time, respectively. With the application of strategy d, *I*_*v*_,  *I*_*hs*_,  *T*_*h*_ and  *I*_*hr*_ within time*t* = 8,10,11 and 30days respectively will be eliminated from the system. This result is a bit more promising than when strategy a and strategy b except possibly strategy c which yielded almost the same results. The control profile shown in Figure 6(g) shows that controls  *u*_1_,  *u*_2_, *u*_3_, and  *u*_4_ decrease from the maximum of 100% to the lower bound. This suggest that a high effort is required for preventive control of drug resistance  *u*_1_, insecticide-treated net  *u*_2_, indoor residual spray (IRS)  *u*_4_, and medical treatment  *u*_3_ of individuals under this strategy.

### 5.2. Cost-Effectiveness Analysis

To analyze the cost-effectiveness of the strategies, we employ the approach of incremental cost-effective ratio (ICER) in [15, 41]. The ICER is used to compare the cost and the health outcomes of two alternative intervention strategies that compete for the same resources.

Based on the values of ICER of the strategy k, the alternative that is more expensive and less ineffective is then excluded. This is done after simulating the optimal control model and then ranking strategies in order of increasing effectiveness measured as the total infection averted. We calculate ICER based on strategy k (*k* = *a*, *b*, *c* *d* ) by using the following formula:

(109) $$\begin{array}{c} \text{ICER }\left(\text{a}\right)=\frac{\text{cost of intervention }\left(\text{a}\right)-\text{cost of intervention }\left(\text{b}\right)}{\text{effect of intervention }\left(\text{a}\right)-\text{effect of intervention }\left(\text{b}\right)}. \end{array}$$

The total infection averted by optimal strategy k during the time period *t*_*f*_ is denoted and defined as

(110) $$\begin{array}{c} \text{T}{\text{A}}_{k}=\frac{A_{1}A_{{kI}_{\text{hs}}}+A_{2}A_{{kI}_{\text{hr}}}+A_{3}A_{{kT}_{h}}+A_{4}A_{{\text{kI}}_{v}}}{A_{1}+A_{2}+A_{3}+A_{4}}, \end{array}$$

where

(111) $$\begin{array}{c} A_{{kI}_{hs}}=t_{f}I_{hs}\left(0\right)-\int_{t_{0}}^{t_{f}}I_{hs}^{**}\left(t\right)dt,\\ A_{{kI}_{hs}}=t_{f}I_{hr}\left(0\right)-\int_{t_{0}}^{t_{f}}I_{hr}^{**}\left(t\right)dt,\\ A_{{kI}_{hs}}=t_{f}T_{h}\left(0\right)-\int_{t_{0}}^{t_{f}}T_{h}^{**}\left(t\right)dt,\\ A_{{kI}_{hs}}=t_{f}I_{v}\left(0\right)-\int_{t_{0}}^{t_{f}}I_{v}^{**}\left(t\right)dt. \end{array}$$

And *A*_*kI*_*hs*__,  *A*_*kI*_*hs*__, *A*_*kI*_*hs*__, and  *A*_*kI*_*v*__ are the total infected humans with drug-sensitive disease parasite strains, infected humans with drug-resistant disease parasite strains, infective in treated human populations, and infected mosquito populations, respectively, averted by optimal strategy k during the time period final time  *t*_*f*_,  *I*_*hs*_^∗∗^, *I*_*hr*_^∗∗^, *T*_*h*_^∗∗^, and *I*_*v*_^∗∗^ that are the optimal solutions associated with optimal controls (*u*_1_^∗^, *u*_2_^∗^, *u*_3_^∗^, *u*_4_^∗^) (49), and *I*_*hs*_(0), *I*_*hr*_(0), *T*_*h*_(0), and *I*_*v*_(0) are the corresponding initial values. Note that these initial values are obtained as the equilibrium proportion of system (49) with no postexposure intervention (*u*_1_ = *u*_2_ = *u*_3_ = *u*_4_ = 0). The total cost associated with a strategy is denoted and given by

(112) $$\begin{array}{c} C_{\text{kT}}=\int_{t_{0}}^{t_{f}}\left[d_{1}u_{1}^{*}\left(t\right)\left(S_{h}^{**}\left(t\right)+I_{\text{hs}}^{**}\left(t\right)+I_{\text{hr}}^{**}\left(t\right)+T_{h}^{**}\left(t\right)\right)+d_{2}u_{2}^{*}\left(t\right)\left(S_{h}^{**}\left(t\right)+I_{\text{hs}}^{**}\left(t\right)+I_{\text{hr}}^{**}\left(t\right)+S_{v}^{**}\left(t\right)+I_{v}^{**}\left(t\right)\right)+d_{3}u_{3}^{*}\left(t\right)\left(S_{h}^{**}\left(t\right)+I_{\text{hs}}^{**}\left(t\right)+T_{h}^{**}\left(t\right)\right)+d_{4}u_{4}^{*}\left(t\right)\left(S_{v}^{**}\left(t\right)+I_{v}^{**}\left(t\right)\right)\right]dt, \end{array}$$

where  *d*_1_ corresponds to the per person unit cost following preventive control of drug resistance intervention,  *d*_2_ corresponds to the per person unit cost of preventive control of ITN intervention, *d*_3_ corresponds to the per person unit cost of treatment intervention, and *d*_4_ corresponds to the per person unit cost of preventive control of IRS intervention. Parameter values from Table 1 are used to estimate the total infection averted and total cost presented in Table 2.

It follows here that after rearranging control strategies in Table 2 in increasing order of effectiveness (TA_*k*_), incremental cost effectiveness ratio ICER for each strategy is computed and given as follows:

(113) $$\begin{array}{c} \text{ICER}\left(\text{b}\right)=\frac{{\Delta C}_{\text{Tb}}}{\mathrm{\Delta T}{\text{A}}_{b}}=\frac{1829200}{3824.77275}=478.2506359365,\\ \text{ICER}\left(\text{a}\right)=\frac{C_{\text{Ta}}-C_{\text{Tb}}}{\text{T}{\text{A}}_{a}-\text{Tb}}=\frac{{\Delta C}_{\text{Ta}}\;}{\mathrm{\Delta T}{\text{A}}_{a}}=4646153.8461538,\\ \text{ICER}\left(\text{c}\right)=\frac{C_{\text{Tc}}-C_{\text{Ta}}}{\text{T}{\text{A}}_{c}-\text{T}{\text{A}}_{a}}=\frac{{\Delta C}_{\text{Tc}}\;}{\mathrm{\Delta T}{\text{A}}_{c}}=-898270270.27027,\\ \text{ICER}\left(\text{d}\right)=\frac{C_{\text{Td}}-C_{\text{Tc}}}{\text{T}{\text{A}}_{d}-\text{T}{\text{A}}_{c}}=\frac{{\Delta C}_{\text{Td}}\;}{\mathrm{\Delta T}{\text{A}}_{d}}=1396962.9629. \end{array}$$

Table 3 incorporates all the four strategies, that is, strategies a, b, c, and d, and corresponding total infection averted during each strategy or effectiveness (TA_*k*_) from Table 2 in increasing order and incremental cost-effectiveness ratio ICER.

Because strategy a is less effective and more costly among the other strategy, we excluded it in Table 4. Thus, Table 4 incorporates only three strategies (that is, strategies b, c, and d) and corresponding total infection averted during each strategy or effectiveness (TA_*k*_) from Table 2 in increasing order and incremental cost effectiveness ratio ICER.

Similarly, because strategy d is less effective and more costly among strategies b, c, and d, we excluded it from Table 5. Thus, Table 5 incorporates only two strategies, that is, strategies b and c, and corresponding total infection averted during each strategy or effectiveness (TA_*k*_) from Table 2 in increasing order and incremental cost effectiveness ratio ICER.

Finally, we conclude that the comparison result reveals that strategy c is cheaper than strategy b. Therefore, strategy c (the use of preventive control of insecticide-treated net (ITN), treatment for infected with drug-sensitive parasite, infective in treatment individuals, and indoor residual spray (IRS)) is the best of all possible strategies due to its more effectiveness and less cost or due to its cost-effectiveness and healthy benefits.

## 6. Discussions and Conclusions

In this study, a nonlinear system of ordinary differential equation model that describes the dynamics of malaria disease transmission is formulated and analyzed. Basic properties of the model, existence of disease-free and endemic equilibrium points, and basic reproduction number of the model are derived and analyzed. From this analysis, we conclude that the basic reproduction number of the model is the threshold parameter between the extinction and persistence of the disease. That is, if the basic reproduction number is less than unity, then the disease-free equilibrium point is both locally and globally asymptotically stable resulting in the disease removing out of the host populations. The endemic equilibrium will also exist if the basic reproduction number is greater than unity. Moreover, existence and necessary condition for forward bifurcation when the basic reproduction number is equal to unity are derived and established. Furthermore, optimal combinations of time-dependent control strategies, that is, prevention of drug resistance, insecticide-treated nets ITN, treatment, and indoor residual spray (IRS), are incorporated to the model. Using optimal control theory of Pontryagins's maximum principle, existence, necessary conditions, and optimality system for the optimal control problem are derived and analyzed.

The optimality system, that is, state system (99) and adjoint system (103) with optimal controls in (105), was solved numerically by applying Runge-Kutta fourth-order schemes. Numerical simulation results of these show that the use of a combination of prevention of drug resistance, insecticide-treated net (ITN), active treatment, and indoor residual spray (IRS) or strategy d performs the best by controlling the disease for the time period of intervention introduced. Moreover, cost-effectiveness analysis using ICER indicates that strategy c is the most optimal cost-effective and efficacious strategy.

Finally, we conclude that the application of optimal combinations of control strategies not only reduces the number populations with malaria symptoms but also reduces the emergence of drug resistant malaria strains as well as the spread of the disease.

## Figures and Tables

**Figure 1:** Flow diagram for the transmission of endemic malaria model.

**Figure 2:** Simulation graph for the basic reproduction number  *R*_0_ versus the force of infection mosquitoes to humans.

**Figure 3:** Simulations of the model showing the effect of preventive control of drug resistance, insecticide-treated net (ITN), and treatment controls.

**Figure 4:** Simulations of the model showing the effect of preventive control of drug resistance, indoor residual spray (IRS), and treatment controls.

**Figure 5:** Simulations of the model showing the effect of insecticide-treated net, indoor residual spray (IRS), and treatment controls.

**Figure 6:** Simulations of the model showing the effect of preventive control of drug resistance, insecticide-treated net, indoor residual spray, and treatment controls.

**Table 1:** Lists of parameters of model system (12).

Parameter symbol	Value	Source
*β*_*h*_	0.8333	[30]
*μ*_*h*_	0.00005447	[31]
*δ*_*h*_	0.0680	[32]
*γ*_*s*_	0.0022	[33]
*γ*_*r*_	0.00019	[34]
*τ*	0.5000	Assumed
*ω*	0.2000	[35]
*ϕ*	0.5020	[35]
*Λ*_*v*_	0.0710	[36]
*δ*_*v*_	0.0100	[37]
*μ*_*v*_	0.0500	[38]
*Λ*_*h*_	0.00000575	[31]
*θ*	0.0167	[39]
*ρ*	0.7000	[40]
*β*_*v*_	0.48	[39]
*β*	0.2500	Assumed
*δ*	0.2500	Assumed
*α*	0.0500	Assumed
*ε*	0.0500	Assumed
*π*	0.5000	Assumed
*σ*_*r*_	0.0500	Assumed

**Table 2:** Cases averted and total costs.

Strategy k	*A*_*kI*_*hs*__	*A*_*kI*_*hr*__	*A*_kT_*h*__	*A*_kI_*v*__	TA_*k*_	Costs ($)*C*_kT_
d	2699.9820	2699.8830	899.9910	8999.9370	3824.94825	2056700
c	2699. 9820	2699.8560	899.9910	8999.9100	3824.93475	1708000
b	2699.955	2699.1810	899.9550	9000.0000	3824.77275	1829200
a	2699. 9820	2699.8650	899.9910	8999.9100	3824.9255	2538900

**Table 3:** Incremental cost-effectiveness ratios of different optimal control strategies.

Strategy k	TA_*k*_	ΔTA_*k*_	Costs ($) *C*_*Tk*_	Δ*C*_Tk_	ICER (Δ*C*_Tk_/ΔTA_*k*_)
b	3824.77275	3824.77275	1829200	1829200	478.2506359365
a	3824.9255	0.15275	2538900	709700	4,646,153.8461538
c	3824.93475	0.00925	1708000	-830900	-898,270,270.27027
d	3824.94825	0.0135	20567000	18859000	1,396,962.9629

**Table 4:** Incremental cost-effectiveness ratios for optimal control strategies b, d, and c.

Strategy k	TA_*k*_	ΔTA_*k*_	Costs ($) *C*_Tk_	Δ*C*_Tk_	ICER (Δ*C*_Tk_/ΔTA_*k*_)
b	3824.77275	3824.77275	1829200	1829200	478.2506359365
c	3824.93475	0.00925	1708000	-830900	-898,270,270.27027
d	3824.94825	0.0135	20567000	18859000	1,396,962.9629

**Table 5:** Incremental cost-effectiveness ratios for optimal control strategies b and c.

Strategy k	TA_*k*_	ΔTA_*k*_	Costs ($) *C*_Tk_	Δ*C*_Tk_	ICER (Δ*C*_Tk_/ΔTA_*k*_)
b	3824.77275	3824.77275	1829200	1829200	478.2506359365
c	3824.93475	0.00925	1708000	-830900	-898,270,270.27027

## Data Availability

In this paper, some parameter values are cited from the previous literatures which are listed in our references. Because of the lack of the available literatures and data, the other parameter values are technically assumed (see details in Table 1).
